# A Mathematical Modeling Analysis of Racism and Corruption Codynamics with Numerical Simulation as Infectious Diseases

**DOI:** 10.1155/2022/9977727

**Published:** 2022-08-11

**Authors:** Belela Samuel Kotola, Shewafera Wondimagegnhu Teklu

**Affiliations:** Department of Mathematics, Natural Science, Debre Berhan University, Debre Berhan, Ethiopia

## Abstract

Racism and corruption are mind infections which affect almost all public and governmental sectors. However, we cannot find enough published literatures on mathematical model analyses of racism and corruption coexistence. In this study, we have contemplated the dynamics of racism and corruption coexistence in communities, using deterministic compartmental model to analyze and suggest proper control strategies to stakeholders. We used qualitative and comprehensive mathematical methods and analyzed both the racism model in the absence of corruption and the corruption model in the absence of racism. We have computed basic reproduction numbers by applying the next generation matrix method. The developed model has a disease-free equilibrium point that is locally asymptotically stable whenever the reproduction number is less than one. Additionally, we have done sensitivity analysis to observe the effect of the parameters on the incidence and transmission of the mind infections that deduce the transmission rates of both the racism and corruption are highly sensitive. The numerical simulation we have simulated showed that the endemic equilibrium point of racism and corruption coexistence model is locally asymptotically stable when max{ *ℛ*_r_, *ℛ*_c_} > 1, the effects of parameters on the basic reproduction numbers, and the effect of parameter on the infectious groups. Finally, the stakeholders must focus on minimizing the transmission rates and increasing the recovery (removed) rate for both racism and corruption action which can be considered prevention and controlling strategies.

## 1. Introduction

Three decades ago, David Mason, a sociologist, who defined the term “institutional racism” would remain a political catchphrase devoid of analytical rigor [1]. Marx and Engels used the term “race” to refer to a wide range of human collectives, including ethnic groups based on skin color, nations, and even social classes [2]. Nowadays, racism is defined as behaviors rooted in beliefs about the innate inferiority of others, scholars working in the Allport tradition argued that racism was more typically expressed as a perception that certain racial groups did not abide by norms of hard work and patriotism and this newer symbolic form of racism has been conceptualized as a set of attitudes acquired through socialization, as perceptions that people teach to each other through interpersonal interaction and learn through education, mass media, religious institutions, and other important sources of communication [3]. Racism is when someone treats another person unfairly because of their membership in a group or because of their opinions about that group's members. It is also when someone has strong negative feelings against another person because of their race [4, 5]. Many of us think that racism is an act of abuse or harassment. However, it does not need to involve brutal or overawing activities. Taking the racial nickname, considering situations, and when people may be ignored by members or participants due to their clan are also racism [4, 6, 7]. Racism in today's society breeds horrible diseases in communities including serious dangers of lingering flaws, confounding of corporate structures, and a decline in the social coherence of present associations [8–10]. Violence is the acyclic act that contains an accumulation of stress and acute violence that can be the heart of racism [5, 6, 11]. Many literatures have been done by scholars on the expansion of racism in the community [5–14].

Corruption is an unpleasant act for communities in general; however, it does not trouble and upset everyone on an equal level. Although corruption is harmful to society as a whole, it frequently has a greater negative impact on existing marginalized groups and is primarily practiced in developing nations [15–17]. The illegal gratitude and abuse of public office for private gain and embezzlement of public funds can be considered corruption [18, 19]. Indeed, it is an infectious activity and dishonest behavior in the body of the society, which seems to be cancer to an economic, social, and political renaissance in the country [20–22]. This illegal act can be conducted by a person or institution entrusted with a position of authority often to acquire inappropriate benefits [21]. The willingness to act of corruption can be offered from either the receptor side or the provider side [15]. The act of corruption is found in every sector of society and can affect a small group of people (petty corruption) or affect part or the entire government (grand corruption) [18, 21]. Even if most countries including Ethiopia have anticorruption policies as well as measures that are being made to eradicate corruption, it still remains a worldwide problem among the communities [15, 23]. People who are unable to receive services they are entitled to without using bribes or contacts have practical difficulties and irritation in their daily lives as a result [24, 25]. Different studies on corruption stated in [15, 18, 22, 26–32] clarify the impact of corruption, economically, socially, and politically among the communities.

Today in our globe, ethnic and racial diversity is increasing rapidly [12, 33]. Those who are already impoverished of opportunities due to racism have a great chance of being exacerbated by corruption [4]. Through our review process, we have adhered that there is a tough kinship between racism and corruption. However, in the current research study, there are only a few studies [34–36] that exhibit and examine the problems due to corruption and racism coexistence in the communities. A solid grasp of mathematics for communities in nations is essential for the advancement of science, technology, and economic growth. This is because mathematics skills are very widely essential in understanding other disciplines including social sciences, engineering, sciences, arts, and outspread to all areas of science, technology as well as business enterprises, and hence, it has been becoming a key in all sciences [37]. Li et al. [38] formulated and analyzed a nonlinear dynamical analysis and optimal control strategies for a new rumor-spreading model with comprehensive interventions. They calculated the basic reproduction number with important biological significance, and the stability of equilibriums is proved. Applying the optimal control theory, the expression of optimal control pairs is obtained. In the simulation part, they examined the optimal control under 11 control strategies and through the data analysis of incremental cost-effectiveness ratio and infection averted ratio of all control strategies and provide a flexible control strategy for the security management department. Teklu and Terefe [37] formulated and analyzed a mathematical model on the dynamics of university students' with animosity towards mathematics with optimal control theory. They have shown that the animosity-free equilibrium point is local and global stability when the basic reproduction number is less than unity, and the animosity-dominance equilibrium points local and global stability whenever the basic reproduction number is greater than unity. They carried out numerical simulations, and from the result, they recommend that prevention and treatment control measures are the best strategies to minimize and possibly to eradicate the animosity-infection throughout the community.

One of the phenomena that can be presented by the mathematical model is the impact and expansion of racism-corruption coexistence among the communities. In this study, we have reviewed a literature done by other scholars to examine the spread and transmission of racism and corruption single existence as infectious diseases with a mathematical modelling approach as stated in [8, 9, 12, 15, 18, 21–23, 27, 28, 30, 31, 39–45], some applied modeling approach for social media addiction [20], and some used modeling approach for violence [6, 7, 10, 11]. However, to the best of our knowledge, no one has developed and analyzed a mathematical model on racism-corruption coexistence among individuals in a given society. Consequently, our newly proposed study contemplates the dynamics of racism and corruption coexistence in communities, using a deterministic compartmental model to analyses and suggests proper control strategies to stakeholders. Therefore, in this newly proposed racism-corruption coexistence model, we are motivated and interested to examine this connection by constructing a mathematical model of racism-corruption coexistence contagion with controlling strategies. The structure of the rest of this study is organized as follows. In Section 2, we describe and formulate the compartmental mathematical model of racism-corruption coexistence.  Section 3 is dedicated to examining model analysis including the equilibrium points, basic reproduction numbers, and the stability analysis of the submodels and the main model.  Section 4 presents sensitivity analysis and numerical simulations. Finally, we carried out discussions and conclusions in Sections 5 and 6, respectively.

## 2. Mathematical Model Formulation

### 2.1. Model Descriptions and Assumptions

We have assumed that all the parameters used in this mode are nonnegative. The recruitment rate entering into the susceptible class is from birth and immigration. Moreover, we have considered that the susceptible individuals are equally likely to be corrupt and/or racialist and the corrupt and/or racialist individual compels susceptible individuals into corruption and/or racism practice(s) as they effectively interact. Upon being recovered, individuals become either susceptible or honest from the act of corruption and/or racism. Using the above basic assumptions and descriptions, we have divided the total population *N* into seven distinct classes. These classes are those individuals who are susceptible to corruption or racism  *S* (*t*), those who are corrupted  C(t), those who stopped corruption *R*_1_(*t*), those who are racist  *R*(*t*), those who stopped racism  *R*_2_(*t*), and those who are both corrupted and racist *C*_1_(*t*) and those who stopped both corruption and racism at the same time *R*_3_(*t*).

The susceptible individuals become corrupted with standard incidence rate given by

(1) $$\begin{array}{c} \lambda_{C}\left(t\right)=\frac{\beta }{N}\left(C\left(t\right)+\omega_{1}C_{1}\left(t\right)\right), \end{array}$$

where  *ω*_1_ ≥ 1  is the modification parameter that increases infectivity and  *β* is the corruption transmission rate. Moreover, we have used the racism mass action incidence rate given by

(2) $$\begin{array}{c} \lambda_{R}\left(t\right)=\alpha \left(R\left(t\right)+\omega_{2}C_{1}\left(t\right)\right), \end{array}$$

where  *ω*_2_ ≥ 1 is the modification parameters that increase infectivity and  *α* is the racism transmission rate.

Using the model assumptions and descriptions stated above, the flow chart of the racism and corruption dynamics is given by

Using Figure 1, the corresponding dynamical system of coexistence transmission dynamics is given by

(3) $$\begin{array}{c} \left.\begin{array}{c} \frac{dS}{dt}=\Lambda +\theta_{2}R_{2}+\theta_{3}R_{3}+\theta_{1}R_{1}-\left(\lambda_{R}+\lambda_{C}+\mu \right)S,\\ \frac{dC}{dt}=\lambda_{C}S+\sigma_{1}C_{1}–\left(\gamma_{1}+{\xi \lambda }_{R}+\mu \right)C,\\ \frac{dR}{dt}=\lambda_{R}S+\sigma_{2}C_{1}-\left({\eta \lambda }_{C}+\gamma_{2}+\mu \right)R,\\ \frac{dC_{1}}{dt}={\eta \lambda }_{C}R+{\xi \lambda }_{R}C-\left(\sigma_{2}+\gamma_{3}+\sigma_{1}+\mu \right)C_{1},\\ \frac{dR_{1}}{dt}=\gamma_{1}C-\left(\theta_{1}+\mu \right)R_{1},\\ \frac{dR_{2}}{dt}=\gamma_{2}R-\left(\theta_{2}+\mu \right)R_{2},\\ \frac{dR_{3}}{dt}=\gamma_{3}C_{1}-\left(\theta_{3}+\mu \right)R_{3}. \end{array}\right\} \end{array}$$

## 3. Qualitative Analysis of the Model (3)

Before we analyze the racism-corruption coexistence model (3), we need to gain some background about the racism submodel and corruption submodel expansion dynamics.

### 3.1. Racism Submodel Analysis

We have derived the mathematical model of racism in the absence of corruption from the full racism and corruption coexistence model by making  *C* = *C*_1_ = , *R*_1_ = *R*_3_ = 0, so that we do have the dynamical system

(4) $$\begin{array}{c} \left.\begin{array}{c} \frac{dS}{dt}=\Lambda +\theta_{2}R_{2}-\left(\lambda_{R}+\mu \right)S,\\ \frac{dR}{dt}=\lambda_{R}S-\left(\gamma_{2}+\mu \right)\text{R},\\ \frac{dR_{2}}{dt}=\gamma_{2}R-\left(\theta_{2}+\mu \right)R_{2}. \end{array}\right\} \end{array}$$

**Theorem 1 (Positivity).**

The solutions  *S*(*t*),  *R*(*t*), and  *R*_2_(*t*) of the racism dynamical system (4) are nonnegative for all time *t* > 0.

**Proof**

Let us define  *τ* = sup{*t* > 0 : *S* (*t*) > 0, *R*(*t*) > 0 and *R*_2_(*t*) > 0}.

Since all, *S*(*t*),  *R*(*t*), and *R*_2_(*t*) are continuous so that we can say *τ* > 0. If *τ* = +∞, then positivity holds. Nevertheless, if  0 < *τ* < +∞, then *S*(*t*) = 0 or (*t*) = 0 *R*_2_(*t*) = 0.

From the first equation of the racism model, we do have *dS*/*dt* = *Λ* + *θ*_2_*R*_2_ − (*λ*_*R*_ + *μ*)*S*. Then, after applying the integrating factor method with some mathematical calculations, we have obtained *S*(*τ*) = *gS*(0) + *g*∫_0_^*τ*^exp^∫(*λ*_*R*_ + *μ*)*dt*^(*πλ* + *θ*_2_*R*_2_)*dt* > 0, where  *g* = exp^−(*μτ* + ∫_0_^*τ*^(*λ*_*R*_ + *μ*))^ > 0, *S*(0) > 0, *R*_2_(t) > 0. Moreover using the definition of  *τ*, the solution  *S*(*τ*) > 0 so that *S*(*τ*) ≠ 0. Using the same procedure all, the solutions of the dynamical system are nonnegative.

#### 3.1.1. Racism-Free Equilibrium Point of the Submodel

Racism-free equilibrium point of the racism model in the absences of corruption is obtained by making the right-hand side of equation is equal to zero providing that the racist class is equal to zero as *R* = 0 which gives following result. *E*_*r*_^0^ = (*S*^*O*^, *R*^*O*^, *R*_2_^0^) = (*Λ*/*μ*, 0, 0).

#### 3.1.2. Reproduction Number of Racism Model in the Absences of Corruption

The reproduction number is the average number of people that become racist because of the entry of one racial person into a completely susceptible population in the absence of intervention. Moreover, reproduction number utilizes to determining the effect of the control measures and to understand the capability of the corruption to disseminate in the entire community when the control strategies are applied [18].

The reproduction number of racism in the absence of corruption model denoted by  *ℛ*_*r*_ which is manipulated by Van den Driesch, Pauline, and James Warmouth next-generation matrix approach [46] is the largest eigenvalue of the next generation matrix *FV*^−1^ = [*∂ℱ*_*i*_( *E*_*r*_^*O*^)/*∂x*_*j*_][*∂ν*_*i*_( *E*_*r*_^*O*^)/*∂x*_*j*_]^−1^, where  *ℱ*_*i*_  is the rate of appearance of new infection in compartment  *i* , *ν*_*i*_  is the transfer of infections from one compartment *i*  to another, and *E*_*r*_^0^ is the disease-free equilibrium point  *E*_*r*_^*O*^ = (*S*^*O*^, *R*^*O*^ *R*_2_^0^) = (*Λ*/*μ*, 0, 0)

The general transmission matrix  *ℱ*_*i*_(*x*) and the transition matrix *𝒱*_*i*_(*x*) are given by

(5) $$\begin{array}{c} \;F_{i}\left(x\right)=\left[\begin{array}{c} \lambda_{R}S\\ 0\\ 0 \end{array}\right]\text{and }V_{i}\left(x\right)=\left[\begin{array}{c} \left(\gamma_{2}+\mu \right)R\\ \left(\theta_{2}+\mu \right)R_{2}-\gamma_{2}R\\ \mu S-\Lambda -\theta_{2}R_{2} \end{array}\right]. \end{array}$$

Then, we have obtained

(6) $$\begin{array}{c} F=\left[\begin{array}{cc} \frac{\Lambda \alpha }{\mu } & 0\\ 0 & 0 \end{array}\right],\text{V}=\left[\begin{array}{cc} \left(\gamma_{1}+\mu \right) & 0\\ -\gamma_{2} & \left(\theta_{2}+\mu \right) \end{array}\right], \end{array}$$

(7) $$\begin{array}{c} FV^{-1}=\left[\begin{array}{cc} \frac{\Lambda \alpha }{\left(\gamma_{2}+\mu \right)\mu } & 0\\ 0 & 0 \end{array}\right]. \end{array}$$

Thus the eigenvalues of *FV*^−1^ are {0, *αΛ*/((*γ*_2_ + *μ*)*μ*)}.

The reproduction number of racism in the absence of corruption model is given by

(8) $$\begin{array}{c} \;R_{r}=\frac{\Lambda \alpha }{\left(\gamma_{2}+\mu \right)\mu }. \end{array}$$

#### 3.1.3. Local Stability of Racism-Free Equilibrium Point

**Theorem 2 .**

The racism-free equilibrium point *E*_*r*_^0^ = (*S*^*O*^, *R*^*O*^ *R*_2_^0^) = (*Λ*/*μ*, 0, 0) of the system (4) is locally asymptotically stable if the reproduction number  *ℛ*_*r*_ < 1, and it is unstable if *ℛ*_*r*_ > 1.

**Proof**

The Jacobean matrix at racism-free equilibrium point is *J*( *E*_*r*_^0^) of the model  (4) given by

(9) $$\begin{array}{c} \text{J}\left(E_{r}^{0}\right)=\left[\begin{array}{ccc} -\mu & 0 & \theta_{2}\\ 0 & \alpha \frac{\Lambda }{\mu }-\left(\gamma_{2}+\mu \right) & 0\\ 0 & \gamma_{2} & -\left(\theta_{2}+\mu \right) \end{array}\right]⟹\left[\begin{array}{ccc} -\mu -\lambda & 0 & \theta_{2}\\ 0 & \alpha \frac{\Lambda }{\mu }-\left(\gamma_{2}+\mu \right)-\lambda & 0\\ 0 & \gamma_{2} & -\left(\theta_{2}+\mu \right)-\lambda \end{array}\right]=0. \end{array}$$

By using Software Wolfram Mathematica, we have the eigenvalues  *λ*_1_ = −*μ*, *λ*_2_ = *α*(*Λ*/*μ*) − (*γ*_2_ + *μ*), and *λ*_3_ = −(*θ*_2_ + *μ*). But *λ*_2_ = *α*(*Λ*/*μ*) − (*γ*_2_ + *μ*) can have the form *λ*_2_ = (*αΛ*/*μ*)((*αΛ*/(*μ*(*γ*_2_ + *μ*))) − 1) = (*αΛ*/*μ*)(*ℛ*_*r*_ − 1). Moreover, *λ*_2_ = (*αΛ*/*μ*)(*ℛ*_*r*_ − 1) < 0 if and only if *ℛ*_*r*_ < 1; hence, all the eigenvalues are negative which implies the racism-free equilibrium point is locally asymptotically stable if and only if *ℛ*_*r*_ < 1; otherwise, it is unstable.

#### 3.1.4. Global Stability of Racism-Free Equilibrium Point

**Theorem 3 .**

The racism-free equilibrium is globally asymptotically stable if *ℛ*_*r*_ < 1.

**Proof**

To prove the global asymptotic stability (GAS) of the racism-free equilibrium point, we have used the method of Lyapunov functions.

We defined a Lyapunov function *l*_1_ such that; *l*_1_ = *aR*, where *a* = *μ*/*αΛ*.

(10) $$\begin{array}{c} \Rightarrow \frac{dl_{1}}{dt}=\frac{\lambda_{R}\mu S}{\alpha \Lambda }-R. \end{array}$$

But we do have *λ*_*R*_ = *αR*  and *N* = *S* + *R* + *R*_1_ = *λ*/*μ*.

(11) $$\begin{array}{c} \Rightarrow \frac{dl_{1}}{dt}\leq \left[\;R_{r}-1\right]\text{R so}\frac{dl_{1}}{dt}<0,\;\text{ if }R_{r}<1. \end{array}$$

Moreover, *dl*_1_/*dt* = 0 if *R* = 0  or *R* = 1. From this fact, we do have (*λ*/*μ*, 0, 0) is the only singleton set in {(*S*, *R*, *R*_1_) ∈ *Ω*_1_ : *dl*_1_/*dt* = 0}. Therefore, by the principle of LaSalle (1976), the racism-free equilibrium point is globally asymptotically stable if *ℛ*_*r*_ < 1.

#### 3.1.5. Existence of Endemic Equilibrium Point of Racism Model in the Absences of Corruption

It is mandatory to be sure about number of endemic equilibrium of the model before investigating the global asymptotic stability of the disease-free equilibrium point (DFE). The endemic equilibrium point of the dynamical system of (4) is solved by making right side of the system equal to zero providing that  *R* ≠ 0. Suppose the endemic equilibrium point of the model is denoted by *E*_*r*_^∗^ = (*S*^∗^, *R*^∗^ *R*_2_^∗^).

The corresponding force of infection is *λ*_*R*_(*t*) = *α*(*R*(*t*)), and we have derived the following:

(12) $$\begin{array}{c} \lambda_{R}=\frac{\alpha \Lambda \lambda_{R}\left(\theta_{2}+\mu \right)}{\left(\lambda_{R}+\mu \right)\left(\theta_{2}+\mu \right)\left(\gamma_{2}+\mu \right)-\theta_{2}\gamma_{2}\lambda_{R}}\Rightarrow \lambda_{R}\left[\left(\lambda_{R}+\mu \right)\left(\theta_{2}+\mu \right)\left(\gamma_{2}+\mu \right)-\theta_{2}\gamma_{2}\lambda_{R}\right]=\alpha \Lambda \lambda_{R}\left(\theta_{2}+\mu \right). \end{array}$$

⇒*λ*_*R*_ = 0 or (*λ*_*R*_ + *μ*)(*θ*_2_ + *μ*)(*γ*_2_ + *μ*) − *θ*_2_*γ*_2_*λ*_*R*_ = *αΛ*(*θ*_2_ + *μ*) after simplification and rearrangement of the terms; we have *λ*_*R*_ = 0 or *λ*_*R*_ = (*γ*_2_ + *μ*)(*θ*_2_ + *μ*)/(*γ*_2_ + *θ*_2_ + *μ*)((*αΛ*/(*μ*(*γ*_2_ + *μ*))) − 1).

(13) $$\begin{array}{c} \Rightarrow \lambda_{R}=0\text{ or }\lambda_{R}=\frac{\left(\gamma_{2}+\mu \right)\left(\theta_{2}+\mu \right)}{\left(\gamma_{2}+\theta_{2}+\mu \right)}\left(R_{r}-1\right)\Rightarrow \lambda_{R}>0,\;\text{if }R_{r}>1. \end{array}$$

Therefore, there is unique endemic equilibrium point for the racism model in the absence of corruption given by *E*_*r*_^∗^ = (*S*^∗^, *R*^∗^, *R*_2_^∗^ ) exist when  *ℛ*_*r*_ > 1 where

(14) $$\begin{array}{c} S^{*}=\frac{\Lambda \left(\theta_{2}+\mu \right)\left(\gamma_{2}+\mu \right)}{\left(\lambda_{R}+\mu \right)\left(\theta_{2}+\mu \right)\left(\gamma_{2}+\mu \right)-\theta_{2}\gamma_{2}\lambda_{R}},\\ R^{*}=\frac{\Lambda \lambda_{R}\left(\theta_{2}+\mu \right)}{\left(\lambda_{R}+\mu \right)\left(\theta_{2}+\mu \right)\left(\gamma_{2}+\mu S\right)-\theta_{2}\gamma_{2}\lambda_{R}},\\ R_{2}^{*}=\frac{\Lambda \gamma_{2}\left(\gamma_{2}+\mu \right)}{\left(\lambda_{R}+\mu \right)\left(\theta_{2}+\mu \right)\left(\gamma_{2}+\mu \right)-\theta_{2}\gamma_{2}\lambda_{R}}. \end{array}$$

**Theorem 4 .**

The racism model in the absence of corruption has a unique endemic equilibrium point whenever  *ℛ*_*r*_ > 1.

**Theorem 5 .**

The endemic equilibrium point  *E*_*r*_^∗^ = (*S*^∗^, *R*^∗^ *R*_2_^∗^)  is locally asymptotically stable if the  *ℛ*_*r*_ > 1, otherwise unstable. To deduce the local stability of the endemic equilibrium point, we use the method of Jacobian matrix and Routh Hurwitz stability criteria. The corresponding Jacobian matrix of the dynamical system at the endemic equilibrium point *E*_*r*_^∗^ = (*S*^∗^, *R*^∗^ *R*_2_^∗^) is

(15) $$\begin{array}{c} J\left(\;E_{r}^{*}\right)=\left[\begin{array}{ccc} -\left(\alpha R^{*}+\mu \right) & -\alpha S^{*} & \theta_{2}\\ \alpha R^{*} & \alpha S^{*}-\left(\gamma_{2}+\mu \right) & 0\\ 0 & \gamma_{2} & -\left(\theta_{2}+\mu \right) \end{array}\right]. \end{array}$$

Then, the characteristic equation of the above Jacobian matrix is given by

(16) $$\begin{array}{c} \left|\begin{array}{ccc} –\left(\alpha R^{*}+\mu \right)-\lambda & -\alpha S^{*} & \theta_{2}\\ \alpha R^{*} & \alpha S^{*}-\left(\gamma_{2}+\mu \right)-\lambda & 0\\ 0 & \gamma_{2} & -\left(\theta_{2}+\mu \right)-\lambda \end{array}\right|=0,\\ \left|\begin{array}{ccc} A-\lambda & \text{B} & \theta_{2}\\ C & D-\lambda & 0\\ 0 & E & F-\lambda \end{array}\right|=0, \end{array}$$

where *A* = –(((*αΛλ*_*R*_(*θ*_2_ + *μ*))/((*λ*_*R*_ + *μ*)(*θ*_2_ + *μ*)(*γ*_2_ + *μ*) − *θ*_2_*γ*_2_*λ*_*R*_)) + *μ*), *B* = −((*αΛ*(*θ*_2_ + *μ*)(*γ*_2_ + *μ*))/((*λ*_*R*_ + *μ*)(*θ*_2_ + *μ*)(*γ*_2_ + *μ*) − *θ*_2_*γ*_2_*λ*_*R*_)), *C* = (*αΛλ*_*R*_(*θ*_2_ + *μ*))/((*λ*_*R*_ + *μ*)(*θ*_2_ + *μ*)(*γ*_2_ + *μ*) − *θ*_2_*γ*_2_*λ*_*R*_), *D* = ((*αΛ*(*θ*_2_ + *μ*)(*γ*_2_ + *μ*))/((*λ*_*R*_ + *μ*)(*θ*_2_ + *μ*)(*γ*_2_ + *μ*) − *θ*_2_*γ*_2_*λ*_*R*_)) − (*γ*_2_ + *μ*), *E* = *γ*_2_, and *F* = −(*θ*_2_ + *μ*).

(17) $$\begin{array}{c} \Rightarrow \left(A-\lambda \right)\left(D-\lambda \right)\left(F-\lambda \right)-BC\left(F-\lambda \right)+\theta_{2}\left(CE\right)=0,\\ \Rightarrow \lambda^{3}-\left(A+D+F\right)\lambda^{2}+\left(AF+DF-BC+AD\right)\lambda +\left(ADF+EC\theta_{2}-BCF\right)=0,\\ \Rightarrow a_{0}\lambda^{3}+a_{1}\lambda^{2}+a_{2}\lambda +a_{3}=0, \end{array}$$

where  *a*_0_ = 1, *a*_1_ = −(*A* + *D* + *F*), *a*_2_ = (*AF* + *DF* − *BC* + *AD*), and *a*_3_ = (*ADF* + *ECθ*_2_ − *BCF*).

But  *a*_0_ = 1 > 0 and *a*_1_ = (−*θ*_2_*γ*_2_*λ*_*R*_/((*λ*_*R*_ + *μ*)(*θ*_2_ + *μ*)(*γ*_2_ + *μ*) − *θ*_2_*γ*_2_*λ*_*R*_))(1 − (*αΛ*/((*γ*_2_ + *μ*)*μ*))).

(18) $$\begin{array}{c} a_{1}=\left(\frac{-\theta_{2}\gamma_{2}\lambda_{R}}{\left(\lambda_{R}+\mu \right)\left(\theta_{2}+\mu \right)\left(\gamma_{2}+\mu \right)-\theta_{2}\gamma_{2}\lambda_{R}}\right)\left(1-R_{r}\right)>0. \end{array}$$

Following the same algebraic manipulation, all the coefficients of the characteristic's polynomial are positives whenever  *ℛ*_*r*_ > 1. Now, we can determine the local stability of endemic equilibrium point by applying the Routh-Hurwitz criteria on *a*_0_*λ*^3^ + *a*_1_*λ*^2^ + *a*_2_*λ* + *a*_3_ = 0.

(19) $$\begin{array}{c} \begin{array}{c} \lambda^{3}\\ \lambda^{2}\\ \lambda^{1}\\ \lambda^{0} \end{array}\left|\begin{array}{cc} a_{0} & a_{2}\\ a_{1} & a_{3}\\ b_{1} & 0\\ {\text{c}}_{1} & 0 \end{array}\right., \end{array}$$

where

(20) $$\begin{array}{c} b_{1}=\frac{-1}{a_{1}}\left|\begin{array}{cc} a_{0} & a_{2}\\ a_{1} & a_{3} \end{array}\right|=\frac{-1}{a_{1}}\left(a_{0}a_{3}-a_{1}a_{2}\right)=b_{1}=\frac{-1}{a_{1}}\left(a_{0}a_{3}-a_{1}a_{2}\right),\\ b_{1}=\frac{-1}{a_{1}}\left(a_{3}-a_{1}a_{2}\right),\\ \Rightarrow b_{1}=\frac{\left(\lambda_{R}+\mu \right)\left(\theta_{2}+\mu \right)\left(\gamma_{2}+\mu \right)+\theta_{2}\gamma_{2}\lambda_{R}}{\theta_{2}\gamma_{2}\lambda_{R}\left(1-R_{r}\right)}\left(\left(\frac{\alpha \Lambda \lambda_{R}\left(\theta_{2}+\mu \right)}{\left(\lambda_{R}+\mu \right)\left(\theta_{2}+\mu \right)\left(\gamma_{2}+\mu \right)-\theta_{2}\gamma_{2}\lambda_{R}}+\mu \right)\frac{\alpha \Lambda \left(\theta_{2}+\mu \right)\left(\gamma_{2}+\mu \right)}{\left(\lambda_{R}+\mu \right)\left(\theta_{2}+\mu \right)\left(\gamma_{2}+\mu \right)-\theta_{2}\gamma_{2}\lambda_{R}}\left(\theta_{2}+\mu \right)\left(\frac{-\theta_{2}\gamma_{2}\lambda_{R}}{\left(\lambda_{R}+\mu \right)\left(\theta_{2}+\mu \right)\left(\gamma_{2}+\mu \right)-\theta_{2}\gamma_{2}\lambda_{R}}\right)\left(\;1-R_{r}\right)\left(\frac{\alpha \Lambda \lambda_{R}\left(\theta_{2}+\mu \right)}{\left(\lambda_{R}+\mu \right)\left(\theta_{2}+\mu \right)\left(\gamma_{2}+\mu \right)-\theta_{2}\gamma_{2}\lambda_{R}}+\mu \right)\right)>0. \end{array}$$

⇒*b*_1_ > 0 if  *ℛ*_*r*_ > 1.

In the same procedure,

(21) $$\begin{array}{c} c_{1}=\frac{-1}{b_{1}}\left|\begin{array}{cc} a_{1} & a_{3}\\ b_{1} & b_{1} \end{array}\right|=\frac{-1}{b_{1}}\left(b_{1}a_{1}-a_{3}b_{1}\right)=\left(a_{3}-a_{1}\right),\\ c_{1}=\left(\frac{\alpha \Lambda \lambda_{R}\left(\theta_{2}+\mu \right)}{\left(\lambda_{R}+\mu \right)\left(\theta_{2}+\mu \right)\left(\gamma_{2}+\mu \right)-\theta_{2}\gamma_{2}\lambda_{R}}+\mu \right)\left(\frac{\alpha \Lambda \left(\theta_{2}+\mu \right)\left(\gamma_{2}+\mu \right)}{\left(\lambda_{R}+\mu \right)\left(\theta_{2}+\mu \right)\left(\gamma_{2}+\mu \right)-\theta_{2}\gamma_{2}\lambda_{R}}\right)\left(\theta_{2}+\mu \right)\left(\frac{-\theta_{2}\gamma_{2}\lambda_{R}}{\left(\lambda_{R}+\mu \right)\left(\theta_{2}+\mu \right)\left(\gamma_{2}+\mu \right)-\theta_{2}\gamma_{2}\lambda_{R}}\right)\left(\;1-R_{r}\right). \end{array}$$

⇒*c*_1_ > 0 if  *ℛ*_*r*_ > 1.

We have observed that the first column of the Routh-Hurwitz array has no sign change; thus, the endemic equilibrium point of the dynamical system is locally asymptotically stable for *ℛ*_*r*_ > 1.

### 3.2. Mathematical Analysis of the Corruption Model in the Absences of Racism

The mathematical model of corruption in the absence of racism is obtained from the full racism and corruption coexistence model (3) by making  *R* = *R*_2_ = *C*_1_ = 0 so that we do have the dynamical system.

(22) $$\begin{array}{c} \left.\begin{array}{c} \frac{dS}{dt}=\Lambda +\theta_{1}R_{1}-\left(\lambda_{C}+\mu \right)S,\\ \frac{dC}{dt}=\lambda_{C}S–\left(\gamma_{1}+\mu \right)C,\\ \frac{dR_{1}}{\text{d}t}=\gamma_{1}C-\left(\theta_{1}+\mu \right)R_{1}. \end{array}\right\} \end{array}$$

**Theorem 6 (Positivity of the submodel solutions).**

The solutions  *S*(*t*),  *C*(*t*), and  *R*_1_(*t*) of the dynamical system of corruption model (22) are nonnegative for all time *t* > 0.

**Proof**

Let us define *τ* = sup{*t* > 0 : *S* (t) > 0, *C*(*t*) > 0, and *R*_1_(*t*) > 0}.

Since all, *S*(*t*),  *C*(*t*), and *R*_1_(*t*) are continuous so that we can say *τ* > 0. If *τ* = +∞, then positivity holds. Nevertheless, if  0 < *τ* < +∞, then  *S*(*t*) = 0 or (*t*) = 0 and *R*_1_(*t*) = 0.

From the first equation of the racism model, we do have *dS*/*dt* = *Λ* + *θ*_1_*R*_1_ − (*λ*_*C*_ + *μ*)*S*.

Then, applying the integrating factor method with some mathematical calculations, we have obtained *S*(*τ*) = *fS*(0) + *f*∫_0_^*τ*^exp^∫(*λ*_*c*_ + *μ*)*dt*^(*Λ* + *θ*_1_*R*_1_)*dt* > 0, where  *f* = exp^−(*μτ* + ∫_0_^*τ*^(*λ*_*c*_ + *μ*))^ > 0, *S*(0) > 0, *R*_1_(t) > 0. Moreover, using the definition of  *τ*, the solution  *S*(*τ*) > 0 so that *S*(*τ*) ≠ 0. Using the same procedure, all the solutions of the dynamical system are nonnegative.

#### 3.2.1. Corruption-Free Equilibrium Point

Corruption-free equilibrium point of the corruption model in the absences of racism is obtained by making the right-hand side of equation equal to zero providing that the corrupted class is equal to zero as *C* = 0 which gives result  *E*_*c*_^*O*^ = (*S*^*O*^, *C*^*O*^, *R*_1_^*O*^) = (*Λ*/*μ*, 0, 0).

#### 3.2.2. Reproduction Number of Corruption Model in the Absences of Racism

The reproduction number of corruption in the absence of racism model denoted by  *ℛ*_*c*_ which is manipulated by next-generation matrix approach [46] is the largest eigenvalue of the next generation matrix  *FV*^−1^ = [(*∂ℱ*_*i*_( *E*_*c*_^*O*^))/*∂x*_*j*_][(*∂ν*_*i*_( *E*_*c*_^*O*^))/*∂x*_*j*_]^−1^, where  *ℱ*_*i*_  is the rate of appearance of new infection in compartment  *i* , *ν*_*i*_  is the transfer of infections from one compartment *i*  to another where 1 ≤ *i*, *j* ≤ *m*, *m* is the number of infected compartments, and *E*_*c*_^0^ is the disease-free equilibrium point *E*^*O*^ = (*S*^*O*^, *C*^*O*^ *R*_1_^*O*^) = (*Λ*/*μ*, 0, 0).

The general transition matrix  *ℱ*_*i*_(*x*) and the transmission matrix  *𝒱*_*i*_(*x*) are given by

(23) $$\begin{array}{c} \;F_{i}\left(x\right)=\left[\begin{array}{c} \lambda_{C}S\\ 0\\ 0 \end{array}\right]\text{and }V_{i}\left(x\right)=\left[\begin{array}{c} \left(\gamma_{1}+\mu \right)R\\ \left(\theta_{1}+\mu \right)R_{1}-\gamma_{1}R\\ \mu S-\Lambda -\theta_{1}R_{1} \end{array}\right]. \end{array}$$

Then, we have obtained

(24) $$\begin{array}{c} F=\left[\begin{array}{cc} \beta & 0\\ 0 & 0 \end{array}\right],\text{V}=\left[\begin{array}{cc} \left(\gamma_{1}+\mu \right) & 0\\ -\gamma_{1} & \left(\theta_{1}+\mu \right) \end{array}\right], \end{array}$$

(25) $$\begin{array}{c} FV^{-1}=\left[\begin{array}{cc} \frac{\beta }{\left(\gamma_{1}+\mu \right)} & 0\\ 0 & 0 \end{array}\right]. \end{array}$$

Thus, the eigenvalues of *FV*^−1^  are {0, *β*/(*γ*_1_ + *μ*)}.

Therefore, the reproduction number of the corruption model in the absence of racism is given by  *ℛ*_*C*_ = *β*/(*γ*_1_ + *μ*).

#### 3.2.3. Local Stability of Corruption-Free Equilibrium Point

**Theorem 7 .**

The racism-free equilibrium point  *E*_*C*_^*O*^ = (*S*^*O*^, *C*^*O*^ *R*_1_^*O*^) = (*Λ*/*μ*, 0, 0) of the system (22) is locally asymptotically stable if the reproduction number  *ℛ*_*c*_ < 1, and it is unstable if *ℛ*_*c*_ > 1.

**Proof**

The Jacobean matrix at corruption-free equilibrium point is *J*( *E*_*c*_^*O*^ ) of the model (3) is given by

(26) $$\begin{array}{c} \text{J}\left(\;{E_{r}}^{O}\right)=\left[\begin{array}{ccc} -\mu & 0 & \theta_{1}\\ 0 & \beta -\left(\gamma_{1}+\mu \right) & 0\\ 0 & \gamma_{1} & -\left(\theta_{1}+\mu \right) \end{array}\right],\\ ⟹\left|\begin{array}{ccc} -\mu -\lambda & 0 & \theta_{1}\\ 0 & \beta -\left(\gamma_{1}+\mu \right)-\lambda & 0\\ 0 & \gamma_{1} & -\left(\theta_{1}+\mu \right)-\lambda \end{array}\right|=0. \end{array}$$

Using Software Wolfram Mathematica, we have obtained the eigenvalues  *λ*_1_ = −*μ*, *λ*_2_ = *β* − (*γ*_1_ + *μ*), and *λ*_3_ = (*θ*_1_ + *μ*).

But *λ*_2_ = *β* − (*γ*_1_ + *μ*) can have the form  *λ*_2_ = (*γ*_2_ + *μ*)((*β*/(*γ*_2_ + *μ*)) − 1) = (*γ*_2_ + *μ*)(*ℛ*_*c*_ − 1). Moreover, *λ*_2_ = (*γ*_2_ + *μ*)(*ℛ*_*c*_ − 1) < 0 if and only if *ℛ*_*c*_ < 1; hence, all the eigenvalues are negative which implies the disease-free equilibrium point is locally asymptotically stable if and only if *ℛ*_*c*_ < 1; otherwise, it is unstable.

#### 3.2.4. Global Stability of Corruption-Free Equilibrium Point

**Theorem 8 .**

The corruption-free equilibrium is globally asymptotically stable if *ℛ*_*c*_ < 1.

**Proof**

To prove the global asymptotic stability (GAS) of the corruption-free equilibrium point, we have used the method of Lyapunov functions.

We defined a Lyapunov function *l*_3_ such that *l*_3_ = *bC*  where *b* = *μ*/*Λ*, ⇒*dl*_3_/*dt* = (*λ*_*C*_*μS*/*Λ*) − *C*.

But we do have *λ*_*C*_ = *βC*/*N* and *N* = *S* + *C* + *R*_2_ = *λ*/*μ* , ⇒*dl*_2_/*dt* ≤ [ *ℛ*_*r*_ − 1]*C*, and thus (*dl*_2_/*dt*) < 0  if  *ℛ*_*c*_ < 1.

Moreover, *dl*_2_/*dt* = 0 if *C* = 0  or  *ℛ*_*c*_ = 1. From this fact, we do have (*λ*/*μ*, 0, 0) is the only singleton set in {(*S*, *C*, *R*_2_) ∈ *Ω* : *dl*_2_/*dt* = 0}. Therefore, by the principle of LaSalle (1976), racism-free equilibrium point is globally asymptotically stable if *ℛ*_*C*_ < 1.

#### 3.2.5. Existence and Uniqueness of Endemic Equilibrium Point of Corruption Model in the Absences of Racism

It is crucial to be sure about the number of endemic equilibrium of the model before investigating the global asymptotic stability of the DFE. The endemic equilibrium point of the dynamical system of (22) is solved by making right side of the system equal to zero providing that  *C* ≠ 0. Suppose the endemic equilibrium point of the model is denoted by *E*_*C*_^∗^ = (*S*^∗^, *C*^∗^ *R*_1_^∗^). The corresponding force of infection is *λ*_*C*_(*t*) = (*β*/*N*)(*C*(*t*)), and we have derived the following.

(27) $$\begin{array}{c} \lambda_{C}=\frac{\beta C}{\left(\left(\gamma_{1}+\mu \right)/\lambda_{C}\right)\left(C\gamma_{1}/\left(\theta_{1}+\mu \right)\right)+C+\left(C\gamma_{1}/\theta_{1}+\mu \right)},\\ \Rightarrow \gamma_{1}\left(\frac{\gamma_{1}+\mu }{\theta_{1}+\mu }\right)+\frac{\gamma_{1}\lambda_{C}}{\theta_{1}+\mu }+\lambda_{C}=\beta . \end{array}$$

After some algebraic simplification and rearrangement of the terms, we have

(28) $$\begin{array}{c} \lambda_{C}=\gamma_{1}\left(\frac{\gamma_{1}+\mu }{\theta_{1}+\mu }\right)\left(\frac{\beta }{\left(\gamma_{2}+\mu \right)}-1\right),\\ \Rightarrow \lambda_{C}=\left(\frac{\gamma_{1}\left(\gamma_{1}+\mu \right)}{\theta_{1}+\mu }\right)\left(R_{C}-1\right). \end{array}$$

Therefore, there is unique endemic equilibrium point for corruption model in the absence of racism given by *E*_*c*_^∗^ = (*S*^∗^, *C*^∗^, *R*_1_^∗^), where

(29) $$\begin{array}{c} \;S^{*}=\frac{\Lambda \left(\theta_{1}+\mu \right)\left(\gamma_{1}+\mu \right)}{\left(\lambda_{C}+\mu \right)\left(\theta_{1}+\mu \right)\left(\gamma_{1}+\mu \right)-\theta_{1}\gamma_{1}\lambda_{C}},\\ C^{*}=\frac{\Lambda \lambda_{C}\left(\theta_{1}+\mu \right)}{\left(\lambda_{C}+\mu \right)\left(\theta_{1}+\mu \right)\left(\gamma_{1}+\mu \right)-\theta_{1}\gamma_{1}\lambda_{C}},\\ R_{1}^{*}=\frac{\Lambda \gamma_{1}\left(\gamma_{1}+\mu \right)}{\left(\lambda_{C}+\mu \right)\left(\theta_{1}+\mu \right)\left(\gamma_{1}+\mu \right)-\theta_{1}\gamma_{1}\lambda_{C}}. \end{array}$$

#### 3.2.6. Local Stability of Endemic Equilibrium Point of the Corruption Model in the Absence of Racism

**Theorem 9 .**

The endemic equilibrium point  *E*_*c*_^∗^ = (*S*^∗^, *C*^∗^ *R*_1_^∗^)  is locally asymptotically stable if the  *ℛ*_*C*_ > 1, otherwise unstable.

**Proof**

See the Appendix.

### 3.3. The Racism and Corruption Coexistence Model Analysis

#### 3.3.1. Basic Properties of the Coexistence Model (3)

The mathematical modeling is the representation of real world phenomena that can be demonstrated by dealing with different quantitative and qualitative attributes. In this newly extended model, we have represented human populations, which cannot be negative. Therefore, we need to show that all the state variables in our model are always nonnegative as well as the solutions of the dynamical system remains positive with positive initial conditions in the bounded region given by *Ω* = {(*S*, *C*, *R*, *C*_1_, *R*_1_, *R*_2_, *R*_3_) ∈ ℝ_+_^7^, *N* ≤ (*Λ*/*μ*)}.

**Theorem 10 (Positivity of the model solutions).**

The solutions  *S*(*t*),  *C*(*t*), *R*(*t*), *C*_1_(*t*), *R*_1_(*t*), *R*_2_(*t*), and *R*_3_(*t*) of the racism and corruption coexistence model (22) are nonnegative for all time *t* > 0.

**Proof**

By defining, *τ* = sup{*t* > 0 : *S* (t) > 0, *C*(*t*) > 0, *R*(*t*) > 0, *C*_1_(*t*) > 0, *R*_1_(*t*) > 0, *R*_2_(*t*) > 0, and *R*_3_(*t*) > 0}.

All *S*(*t*),  *C*(*t*), *R*(*t*), *C*_1_(*t*), *R*_1_(*t*), *R*_2_(*t*), and *R*_3_(*t*) are continuous so that we can deduce that  *τ* > 0. If *τ* = +∞, then positivity holds. However, if  0 < *τ* < +∞, then  *S*(*t*) = 0 or  *C*(*t*) = 0 or *R*(*t*) = 0 or *C*_1_(*t*) = 0  or  *R*_1_(*t*) = 0 or  *R*_2_(*t*) = 0 or *R*_3_(*t*) = 0.

From the first equation of the racism and corruption coexistence model, we do have *dS*/*dt* = *Λ* + *θ*_2_*R*_2_ + *θ*_3_*R*_3_ + *θ*_1_*R*_1_ − (*λ*_*R*_ + *λ*_*C*_ + *μ*)*S*, and applying the integrating factor method and after some calculations, we have obtained *S*(*τ*) = *hS*(0) + *h*∫_0_^*τ*^exp^∫(*λ*_*R*_ + *λ*_*C*_ + *μ*))*dt*^(*Λ* + *θ*_2_*R*_2_ + *θ*_3_*R*_3_ + *θ*_1_*R*_1_)*dt* > 0, where  *h* = exp^−(*μτ* + ∫_0_^*τ*^(*λ*_*R*_ + *λ*_*C*_ + *μ*))^ > 0,  *S*(0) > 0,  *R*_2_(*t*) > 0,  *R*_3_(*t*) > 0  and  *R*_1_ > 0. Finally, using the definition of  *τ*, the solution  *S*(*τ*) > 0 so that *S*(*τ*) ≠ 0.

Following the same procedure all the solutions of the dynamical system are nonnegative.

**Theorem 11 (Boundedness of the model solutions).**

The region $\Omega =\left\{\begin{array}{c} \left(S,C,R,C_{1},R_{1},R_{2},R_{3}\right)\in {\mathbb{R}}_{+}^{7},N\leq \left(\Lambda /\mu \right) \end{array}\right\}$ is bounded in ℝ_+_^7^.

**Proof**

Since all the state variables are nonnegative in the absence of infections, we have obtained  (*dN*/*dt*) ≤ *Λ* − *μN*. By incorporating standard comparison theorem, we have obtained ∫(*dN*/(*Λ* − *μN*)) ≤ ∫*dt* and integrating both sides gives −1/*μ*ln(*Λ* − *μN*) ≤ *t* + *c*, where *c* is some constant, and after some mathematical calculations and simplifications, we have obtained 0 ≤ *N* (*t*) ≤ (*Λ*/*μ*). This result implies all the possible solutions of the given dynamical system with positive initial conditions are bounded.

#### 3.3.2. Racism and Corruption-Free Equilibrium Point of the Model (3)

The racism and corruption-free equilibrium point of the model is obtained by making the right-hand side of the system (3) is equal to zero providing that all the infected classes are zero as *C* = *R* = *C*_1_ = 0 given by *E*^0^ = (*S*^0^, *C*^0^, *R*^0^, *C*_1_^0^, *R*_1_^0^, *R*_2_^0^, *R*_3_^0^) = (*Λ*/*μ*, 0, 0, 0, 0, 0, 0).

#### 3.3.3. Basic Reproduction Number of the Coexistence Model (3)

The reproduction number of racism and corruption coexistence model denoted by  *ℛ*_*cr*_ the Van den Driesch, Pauline, and James Warmouth next-generation matrix approach [46] is the largest eigenvalue of the next generation matrix  *FV*^−1^ = [*∂ℱ*_*i*_(*E*^*O*^)/*∂x*_*j*_][*∂ν*_*i*_(*E*^*O*^)/*∂x*_*j*_]^−1^, where  *ℱ*_*i*_  is the rate of appearance of new infection in compartment  *i* , *ν*_*i*_  is the transfer of infections from one compartment *i*  to another where 1 ≤ *i*, *j* ≤ *m*, *m* is the number of infected compartments, and *E*_*ch*_^0^ is the disease-free equilibrium point *E*^*O*^ = (*S*^0^, *C*^0^, *R*^0^, *C*_1_^0^, *R*_1_^0^ *R*_2_^0^, *R*_3_^0^) = (*Λ*/*μ*, 0, 0, 0, 0, 0, 0).

The general transmission matrix  *ℱ*_*i*_(*x*) and the transition matrix  *𝒱*_*i*_(*x*) are given by

(30) $$\begin{array}{c} \;F_{i}\left(x\right)=\left[\begin{array}{c} \lambda_{C}S\\ \lambda_{R}S\\ 0\\ 0\\ 0\\ 0 \end{array}\right]\text{ and }V_{i}\left(x\right)=\left[\begin{array}{c} \left(\gamma_{1}+{\xi \lambda }_{R}+\mu \right)C-\sigma_{1}C_{1}\\ \left({\eta \lambda }_{C}+\gamma_{2}+\mu \right)R-\sigma_{2}C_{1}\\ \left(\sigma_{2}+\gamma_{3}+\sigma_{1}+\mu \right)C_{1}-\eta \lambda_{C}R-{\xi \lambda }_{R}C\\ \left(\theta_{1}+\mu \right)R_{1}-\gamma_{1}C\\ \left(\theta_{2}+\mu \right)R_{2}-\gamma_{2}R\\ \left(\theta_{3}+\mu \right)R_{3}-\gamma_{3}C_{1} \end{array}\right]. \end{array}$$

Then, after some calculations, we have obtained

(31) $$\begin{array}{c} F=\left[\begin{array}{ccc} \beta & 0 & \beta \omega_{1}\\ 0 & \frac{\Lambda \alpha }{\mu } & \frac{\Lambda \alpha \omega_{2}}{\mu }\\ 0 & 0 & 0 \end{array}\right],V=\left[\begin{array}{ccc} \left(\gamma_{1}+\mu \right) & 0 & -\sigma_{1}\\ 0 & \left(\gamma_{2}+\mu \right) & -\sigma_{2}\\ 0 & 0 & \left(\sigma_{2}+\gamma_{3}+\sigma_{1}+\mu \right) \end{array}\right],\\ FV^{-1}=\left[\begin{array}{ccc} \frac{\beta }{A} & 0 & -\frac{B\beta \omega_{1}}{AE}\\ 0 & \frac{\Lambda \alpha }{C\mu } & -\frac{D\Lambda \alpha \lambda \omega_{2}}{CE\mu }\\ 0 & 0 & 0 \end{array}\right], \end{array}$$

where  *A* = (*γ*_1_ + *μ*), *B* = −*σ*_1_, *C* = (*γ*_2_ + *μ*), *D* = −*σ*_2_, and *E* = (*σ*_2_ + *γ*_3_ + *σ*_1_ + *μ*).

The eigenvalues of *FV*^−1^  are {0, *αΛ*/(*γ*_2_ + *μ*)*μ*, *β*/(*γ*_1_ + *μ*)}. Thus, the reproduction number of racism and corruption coexistence denoted by  *ℛ*_*rc*_ and is max {*Λα*/(*γ*_2_ + *μ*)*μ*, *β*/(*γ*_1_ + *μ*)}.

That means  *ℛ*_*rc*_ = max{ *ℛ*_*r*_, *ℛ*_*c*_} = max{*Λα*/(*γ*_2_ + *μ*)*μ*, *β*/(*γ*_1_ + *μ*)}.

#### 3.3.4. Local Stability of Coexistence-Free Equilibrium Point of the Model (3)

**Theorem 12 .**

The racism and corruption free equilibrium point *E*^*O*^ = (*S*^*O*^, *C*^*O*^, *R*^*O*^, *C*_1_^*O*^, *R*_1_^*O*^, *R*_2_^*O*^, *R*_3_^*O*^) = (*Λ*/*μ*, 0, 0, 0, 0, 0, 0) of the model is locally asymptotically stable if the reproduction number  *ℛ*_*rc*_ < 1, and it is unstable if *ℛ*_*rc*_ > 1.

**Proof**

The Jacobean matrix  *J*(*X* ) of the model (3) is given by

(32) $$\begin{array}{c} J\left(X\right)=\left[\begin{array}{ccccccc} -\left(\lambda_{R}+\lambda_{C}+\mu \right) & \frac{-\beta }{N}S & -\alpha S & \frac{-\omega_{1}\beta }{N}S-\omega_{1}\alpha S & \theta_{1} & \theta_{2} & \theta_{3}\\ \lambda_{C} & \frac{\beta }{N}S–\left(\gamma_{1}+{\xi \lambda }_{R}+\mu \right) & -\xi \alpha C & \sigma_{1} & 0 & 0 & 0\\ \lambda_{R} & -\frac{\beta }{N}\eta R & \alpha S-\left({\eta \lambda }_{C}+\gamma_{2}+\mu \right) & \sigma_{2} & 0 & 0 & 0\\ 0 & \frac{\beta \eta R}{N}+{\xi \lambda }_{R} & {\eta \lambda }_{C}+\xi \alpha C & -\left(\sigma_{2}+\gamma_{3}+\sigma_{1}+\mu \right) & 0 & 0 & 0\\ 0 & \gamma_{1} & 0 & 0 & -\left(\theta_{1}+\mu \right) & 0 & 0\\ 0 & 0 & \gamma_{2} & 0 & 0 & -\left(\theta_{2}+\mu \right) & 0\\ 0 & 0 & 0 & \gamma_{3} & 0 & 0 & -\left(\theta_{3}+\mu \right) \end{array}\right],\\ ⟹J\left(E^{O}\right)=\left[\begin{array}{ccccccc} -\mu & -\beta & -\alpha \frac{\pi \lambda }{\mu } & -\left(\omega_{1}\beta +\omega_{1}\alpha \right)\frac{\pi \lambda }{\mu } & \theta_{1} & \theta_{2} & \theta_{3}\\ 0 & \beta –\left(\gamma_{1}+\mu \right) & 0 & \sigma_{1} & 0 & 0 & 0\\ 0 & 0 & \alpha \frac{\pi \lambda }{\mu }-\left(\gamma_{2}+\mu \right) & \sigma_{2} & 0 & 0 & 0\\ 0 & 0 & 0 & -\left(\sigma_{2}+\gamma_{3}+\sigma_{1}+\mu \right) & 0 & 0 & 0\\ 0 & \gamma_{1} & 0 & 0 & -\left(\theta_{1}+\mu \right) & 0 & 0\\ 0 & 0 & \gamma_{2} & 0 & 0 & -\left(\theta_{2}+\mu \right) & 0\\ 0 & 0 & 0 & \gamma_{3} & 0 & 0 & -\left(\theta_{3}+\mu \right) \end{array}\right]. \end{array}$$

Using Wolfram Mathematica, we have obtained the eigenvalues of *J*(*E*^*O*^) as *λ*_1_ = −*μ*, *λ*_2_ = *β*–(*γ*_1_ + *μ*), *λ*_3_ = *α*(*πλ*/*μ*) − (*γ*_2_ + *μ*), *λ*_4_ = −(*σ*_2_ + *γ*_3_ + *σ*_1_ + *μ*), *λ*_5_ = −(*θ*_1_ + *μ*),  *λ*_6_ = −(*θ*_2_ + *μ*), *λ*_7_ = −(*θ*_3_ + *μ*).

But *λ*_2_ and *λ*_3_  can be rewritten as follows: *λ*_2_ = *β*–(*γ*_1_ + *μ*) = (*γ*_1_ + *μ*)((*β*/(*γ*_1_ + *μ*)) − 1) and *λ*_3_ = *α*(*Λ*/*μ*) − (*γ*_2_ + *μ*) = (*γ*_2_ + *μ*)((*Λα*/(*γ*_2_ + *μ*)*μ*) − 1).

Hence, all the eigenvalues are negative if  *ℛ*_*rc*_ < 1. Therefore, the racism and corruption coexistence free equilibrium point is locally asymptotically stable if and only if *ℛ*_*rc*_ < 1; otherwise, it is unstable.

#### 3.3.5. Existence of Racism-Corruption Coexistence Equilibrium Point

The racism-corruption coexistence endemic equilibrium point of the full model (3) is denoted by *E*^∗^ = (*S*^∗^, *C*^∗^, *R*^∗^, *C*_1_^∗^, *R*_1_^∗^, *R*_2_^∗^, *R*_3_^∗^) which occurs when the mind infection persist in the community, and we computed by making the right hand side of the model as zero and obtained as

(33) $$\begin{array}{c} S^{*}=\frac{\Lambda +\theta_{1}R_{1}^{*}+\theta_{2}R_{2}^{*}+\theta_{3}R_{3}^{*}}{\left(\lambda_{R}^{*}+\lambda_{C}^{*}+\mu \right)},C^{*}=\frac{\lambda_{C}^{*}S^{*}+\sigma_{1}C_{1}^{*}}{\left(\gamma_{1}+\xi \lambda_{R}^{*}+\mu \right)},C_{1}^{*}=\frac{\eta \lambda_{C}^{*}R^{*}+\xi \lambda_{R}^{*}C^{*}}{\left(\sigma_{2}+\gamma_{3}+\sigma_{1}+\mu \right)},\\ R^{*}=\frac{\lambda_{R}^{*}S^{*}+\sigma_{2}C_{1}^{*}}{\left(\eta \lambda_{C}^{*}+\gamma_{2}+\mu \right)},R_{1}^{*}=\frac{\gamma_{1}C^{*}}{\left(\theta_{1}+\mu \right)},R_{2}^{*}=\frac{\gamma_{2}R^{*}}{\left(\theta_{2}+\mu \right)},R_{3}^{*}=\frac{\gamma_{3}C_{1}^{*}}{\left(\theta_{3}+\mu \right)}. \end{array}$$

From the analysis of the corruption only submodel (22) and the racism only submodel (4), we have shown that there is no endemic equilibrium point if *ℛ*_*c*_ < 1  and *ℛ*_*r*_ < 1, respectively, implying that there is no endemic equilibrium point if *ℛ*_*rc*_ < 1 for the coexistence model (3); in other words, the racism-corruption coexistence free equilibrium point is globally stable if *ℛ*_*rc*_ < 1.

The summary of the racism-corruption mind infection persistence equilibrium points: The explicit computation of the mind infection persistence equilibrium point of the coinfection model (3) in terms of model parameters is difficult analytically since the system is highly nonlinear; however, the model (3) endemic equilibriums corresponds to

1. *E*_1_^∗^ = (*S*^∗^, 0, *R*^∗^, 0, *R*_1_^∗^, 0, 0), if  *ℛ*_*r*_ > 1 is the corruption-free (racism persistence) equilibrium point. The analysis of the equilibrium *E*_1_^∗^ is similar to the endemic equilibrium *E*_*r*_^∗^ in the model (2)
2. *E*_2_^∗^ = (*S*^∗^, *C*^∗^, 0, 0, 0, *R*_2_^∗^, 0), if *ℛ*_*c*_ > 1 is the racism-free (corruption persistence) equilibrium point. The analysis of the equilibrium *E*_2_^∗^ is similar to the endemic equilibrium *E*_*c*_^∗^ in equations (3)
3. *E*_*rc*_^∗^ = (*S*^∗^, *C*^∗^, *R*^∗^, *C*_1_^∗^, *R*_1_^∗^, *R*_2_^∗^, *R*_3_^∗^) is the racism-corruption coexistence persistence equilibrium point

#### 3.3.6. Bifurcation Analysis of the Racism-Corruption Coexistence Model

In this section, we apply the center manifold theory given by Theorem 2 of Castillo-Chavez and Song [47] to ascertain the local asymptotic stability of the endemic equilibrium due to the convolution of the first approach (eigenvalues of the Jacobian). To make use of the center manifold theory, the following change of variables is made by symbolizing:  *S* = *x*_1_, *C* = *x*_2_, *R* = *x*_3_, *C*_1_ = *x*_4_, and *R*_1_ = *x*_5_, *R*_2_ = *x*_6_, and *R*_3_ = *x*_7_ such that  *N* = *x*_1_ + *x*_2_ + *x*_3_ + *x*_4_ + *x*_5_ + *x*_6_ + *x*_7_. Furthermore, by using vector notation  *X* = (*x*_1_, *x*_2_, *x*_3_, *x*_4_, *x*_5_, *x*_6_, *x*_7_)^*T*^, the Racism-Corruption coexistence model (3) can be written in the form *dX*/*dt* = *F*(*X*) with *F* = (*f*_1_, *f*_2_, *f*_3_, *f*_4_, *f*_5_, *f*_6_, *f*_7_)^*T*^, as follows:

(34) $$\begin{array}{c} \frac{{dx}_{1}}{dt}=f_{1}=\Lambda +\theta_{1}x_{5}+\theta_{2}x_{6}+\theta_{3}x_{7}-\left(\lambda_{R}+\lambda_{C}+\mu \right)x_{1}, \end{array}$$

(35) $$\begin{array}{c} \frac{{dx}_{2}}{dt}=f_{2}=\lambda_{C}x_{1}+\sigma_{1}x_{4}–\left(\gamma_{1}+{\xi \lambda }_{R}+\mu \right)x_{2}, \end{array}$$

(36) $$\begin{array}{c} \frac{dx_{4}}{dt}={\eta \lambda }_{C}x_{3}+{\xi \lambda }_{R}x_{2}-\left(\sigma_{2}+\gamma_{3}+\sigma_{1}+\mu \right)x_{4}, \end{array}$$

(37) $$\begin{array}{c} \frac{dx_{5}}{dt}=\gamma_{1}x_{2}-\left(\theta_{1}+\mu \right)x_{5}, \end{array}$$

(38) $$\begin{array}{c} \frac{dx_{6}}{dt}=\gamma_{2}x_{3}-\left(\theta_{2}+\mu \right)x_{6}, \end{array}$$

with *λ*_*R*_ = *α*(*x*_3_ + *ω*_2_*x*_4_) and *λ*_*C*_ = (*β*/*N*)(*x*_2_ + *ω*_1_*x*_4_).

Then, the method entails evaluating the Jacobian of the system (34) at the DFE point  *E*_*CR*_^0^, denoted by *J*(*E*_*CR*_^0^), and this gives us

(39) $$\begin{array}{c} J\left(\;E_{CR}^{0}\right)=\left(\begin{array}{ccccccc} -\mu & -\beta & -\alpha x_{1}^{0} & -\beta \omega_{1}+\alpha \omega_{2}x_{1}^{0} & \theta_{1} & \theta_{2} & \theta_{3}\\ 0 & \;\beta -\left(\gamma_{1}+\mu \right) & 0\; & \beta \omega_{1}+\sigma_{1} & 0 & 0 & 0\\ \;0 & 0 & \alpha x_{1}^{0}-\left(\gamma_{2}+\mu \right) & \alpha \omega_{2}x_{1}^{0}+\sigma_{2} & 0 & 0 & 0\\ 0 & 0 & 0 & -\left(\sigma_{2}+\gamma_{3}+\sigma_{1}+\mu \right) & 0 & 0 & 0\\ 0 & \gamma_{1} & 0 & 0 & -\left(\theta_{1}+\mu \right) & 0 & 0\\ 0 & 0 & \gamma_{2} & 0 & 0 & \left(\theta_{2}+\mu \right) & 0\\ 0 & 0 & 0 & \gamma_{3} & 0 & 0 & \left(\theta_{3}+\mu \right) \end{array}\right). \end{array}$$

Consider *ℛ*_*CR*_ = 1, and suppose that *β* = *β*^∗^ is chosen as a bifurcation parameter.

From *ℛ*_*CR*_ = 1 as  *ℛ*_*CR*_ = *β*/(*γ*_1_ + *μ*) = 1 and solving for *β*, we have obtained *β* = *β*^∗^ = *γ*_1_ + *μ*.

(40) $$\begin{array}{c} J_{\beta^{*}}=\left(\begin{array}{ccccccc} -\mu & -\beta^{*} & -\alpha x_{1}^{0} & -\beta^{*}\omega_{1}+\alpha \omega_{2}x_{1}^{0} & \theta_{1} & \theta_{2} & \theta_{3}\\ 0 & \;\beta^{*}-\left(\gamma_{1}+\mu \right) & 0\; & \beta \omega_{1}+\sigma_{1} & 0 & 0 & 0\\ \;0 & 0 & \alpha x_{1}^{0}-\left(\gamma_{2}+\mu \right) & \alpha \omega_{2}x_{1}^{0}+\sigma_{2} & 0 & 0 & 0\\ 0 & 0 & 0 & -\left(\sigma_{2}+\gamma_{3}+\sigma_{1}+\mu \right) & 0 & 0 & 0\\ 0 & \gamma_{1} & 0 & 0 & -\left(\theta_{1}+\mu \right) & 0 & 0\\ 0 & 0 & \gamma_{2} & 0 & 0 & -\left(\theta_{2}+\mu \right) & 0\\ 0 & 0 & 0 & \gamma_{3} & 0 & 0 & -\left(\theta_{3}+\mu \right) \end{array}\right). \end{array}$$

After some steps of the calculation, we have obtained the eigenvalues of *J*_*β*^∗^_ as *λ*_1_ = −*μ*, *λ*_2_ = 0 or *λ*_3_ = *αx*_1_^0^ − (*γ*_2_ + *μ*) = *αΛ*/*μ* − (*γ*_2_ + *μ*) = (*γ*_2_ + *μ*)[(*αΛ*/*μ*(*γ*_2_ + *μ*)) − 1] = (*γ*_2_ + *μ*)[ *ℛ*_*R*_ − 1] < 0  if  *ℛ*_*R*_ < 1  or *λ*_4_ = −(*σ*_2_ + *γ*_3_ + *σ*_1_ + *μ*) or *λ*_5_ = −(*θ*_1_ + *μ*) or *λ*_6_ = −(*θ*_2_ + *μ*), and *λ*_7_ = −(*θ*_3_ + *μ*).

It follows that the Jacobian *J*(*E*_*CR*_^0^) of equation (34) at the disease-free equilibrium with *β* = *β*^∗^, denoted by *J*_*β*^∗^_, has a simple zero eigenvalue with all the remaining eigenvalues have negative real part. Hence, the Centre Manifold theory given by Theorem 2 of Castillo-Chavez and Song [47] can be used to analyze the dynamics of the model (3). In particular, it will be used to show that the model (34) undergoes backward bifurcation at *ℛ*_*CR*_ = 1.

In eigenvectors of  *J*_*β*^∗^_, for the case  *ℛ*_*CR*_ = 1, it can be shown that the Jacobian of the system (34) at *β* = *β*^∗^ (denoted by *J*_*β*^∗^_) has right eigenvectors associated with the zero eigenvalue given by *u* = (*u*_1_, *u*_2_, *u*_3_, *u*_4_, *u*_5_, *u*_6_, *u*_7_)^*T*^ as

(41) $$\begin{array}{c} \left(\begin{array}{ccccccc} -\mu & -\beta^{*} & -\alpha x_{1}^{0} & M_{1} & \theta_{1} & \theta_{2} & \theta_{3}\\ 0 & \;\beta^{*}-\left(\gamma_{1}+\mu \right) & 0\; & \beta +\sigma_{1} & 0 & 0 & 0\\ \;0 & 0 & M_{2} & \alpha \omega_{2}x_{1}^{0}+\sigma_{2} & 0 & 0 & 0\\ 0 & 0 & 0 & M_{3} & 0 & 0 & 0\\ 0 & \gamma_{1} & 0 & 0 & -\left(\theta_{1}+\mu \right) & 0 & 0\\ 0 & 0 & \gamma_{2} & 0 & 0 & -\left(\theta_{2}+\mu \right) & 0\\ 0 & 0 & 0 & \gamma_{3} & 0 & 0 & -\left(\theta_{3}+\mu \right) \end{array}\right)\left(\begin{array}{c} u_{1}\\ u_{2}\\ u_{3}\\ u_{4}\\ u_{5}\\ u_{6}\\ u_{7} \end{array}\right)=\left(\begin{array}{c} 0\\ 0\\ 0\\ 0\\ 0\\ 0\\ 0 \end{array}\right), \end{array}$$

where *M*_1_ = −*β*^∗^*ω*_1_ − *αω*_2_*x*_1_^0^, *M*_2_ = *αx*_1_^0^ − (*γ*_2_ + *μ*), and *M*_3_ = −(*σ*_2_ + *γ*_3_ + *σ*_1_ + *μ*).

Then solving equation (41) the right eigenvectors associated with the zero eigenvalue are given by

(42) $$\begin{array}{c} u_{1}=-\frac{\left(\theta_{1}+\mu \right)\beta^{*}u_{2}+\theta_{1}\gamma_{1}u_{2},}{\mu \left(\theta_{1}+\mu \right)}<0,u_{2}=u_{2}>0,\\ u_{3}=0,u_{4}=0,u_{5}=\frac{\gamma_{1}}{\left(\theta_{1}+\mu \right)}u_{2}>0,u_{6}=0,u_{7}=0. \end{array}$$

Similarly, the left eigenvector associated with the zero eigenvalues at *β* = *β*^∗^ given by *v* = (*v*_1_, *v*_2_, *v*_3_, *v*_4_, *v*_5_, *v*_6_, *v*_7_)^*T*^ as

(43) $$\begin{array}{c} {\left(\begin{array}{c} v_{1}\\ v_{2}\\ v_{3}\\ v_{4}\\ v_{5}\\ v_{6}\\ v_{7} \end{array}\right)}^{T}*\left(\begin{array}{ccccccc} -\mu & \beta^{*} & \alpha x_{1}^{0} & M_{1} & \theta_{1} & \theta_{2} & \theta_{3}\\ 0 & \;\beta^{*}-\left(\gamma_{1}+\mu \right) & 0\; & \beta +\sigma_{1} & 0 & 0 & 0\\ \;0 & 0 & M_{2} & \alpha \omega_{2}x_{1}^{0}+\sigma_{2} & 0 & 0 & 0\\ 0 & 0 & 0 & M_{3} & 0 & 0 & 0\\ 0 & \gamma_{1} & 0 & 0 & -\left(\theta_{1}+\mu \right) & 0 & 0\\ 0 & 0 & \gamma_{2} & 0 & 0 & \left(\theta_{2}+\mu \right) & 0\\ 0 & 0 & 0 & \gamma_{3} & 0 & 0 & \left(\theta_{3}+\mu \right) \end{array}\right)=\left(\begin{array}{c} 0\\ 0\\ 0\\ 0\\ 0\\ 0\\ 0\\ 0 \end{array}\right). \end{array}$$

Then, solving equation (43) the left eigenvectors associated with the zero eigenvalue are given by

(44) $$\begin{array}{c} v_{1}=v_{3}=v_{4}=v_{5}=v_{6}=v_{7}=0\text{ and }v_{2}=v_{2}>0. \end{array}$$

After some steps of calculations, the bifurcation coefficients *a* and *b* are obtained as

(45) $$\begin{array}{c} a=\overset{7}{\underset{i,j,k=1}{\sum }}v_{2}u_{i}u_{j}\frac{\partial^{2}f_{2}}{\partial x_{i}\partial x_{j}}=2v_{2}u_{1}u_{2}\frac{\partial^{2}f_{2}}{\partial x_{1}\partial x_{2}}+2v_{2}u_{3}u_{2}\frac{\partial^{2}f_{2}}{\partial x_{3}\partial x_{2}}=2v_{2}u_{2}\left[u_{1}\frac{\partial^{2}f_{2}}{\partial x_{1}\partial x_{2}}+u_{3}\frac{\partial^{2}f_{2}}{\partial x_{3}\partial x_{2}}\right]<2v_{2}u_{2}\left[u_{1}\beta +\xi \alpha u_{3}\right]=-2v_{2}u_{2}\left[\frac{\beta \left(\theta_{1}+\mu \right)\beta^{*}u_{2}+\theta_{1}\gamma_{1}u_{2},}{\mu \left(\theta_{1}+\mu \right)}\right]<0. \end{array}$$

Thus, the coefficient  *a* is negative.

Moreover,

(46) $$\begin{array}{c} b=\overset{7}{\underset{i,k=1}{\sum }}v_{k}u_{i}\frac{\partial^{2}f_{k}}{\partial x_{i}\partial \beta }\left(E_{CR}^{0}\right)=\overset{7}{\underset{i=1}{\sum }}v_{2}u_{i}\frac{\partial^{2}f_{2}}{\partial x_{i}\partial \beta }=v_{2}u_{2}\frac{\partial^{2}f_{2}}{\partial x_{2}\partial \beta }={\beta v}_{2}u_{2}>0. \end{array}$$

Since *u*_2_ > 0 and *v*_2_ > 0 then *a* < 0 and *b* > 0, the Racism-Corruption coexistence model (3) exhibits the forward bifurcation, which occurs at  *ℛ*_*CR*_ = 1. That is, if  *ℛ*_*CR*_ < 1, then there is no occurrence of coexistence endemic equilibrium and the coexistence free equilibrium is the only local attractor. But if  *ℛ*_*CR*_ > 1, then the coexistence endemic equilibrium exists. For this reason, there is a forward bifurcation because in the neighborhood of the bifurcation point, the coexistence mind infection prevalence is an increasing function of  *ℛ*_*CR*_. Hence, from in Castillo-Chavez and Song [47], the Racism-Corruption coexistence model (3) endemic equilibrium is locally asymptotically stable whenever  *ℛ*_*CR*_ > 1.

## 4. Sensitivity Analysis and Numerical Simulations

### 4.1. Sensitivity Analysis

The normalized forward sensitivity index of a variable racism and corruption coexistence model (3) basic reproduction number denoted by the symbol  *ℛ*_*rc*_  that is differentiable with a parameter *ε*  is defined as SI (*p*) = (*∂ℛ*_*rc*_/*∂ε*)∗(*ε*/*ℛ*_*rc*_)  as stated in literatures [48–50].

The sensitivity indices enable us to examine the relative importance of different parameters in racism and corruption incidence and prevalence. The most sensitive parameter has the magnitude of the sensitivity index larger than that of all other parameters. We can calculate the sensitivity index in terms of *ℛ*_*r*_  and *ℛ*_*c*_  since *ℛ*_*rc*_ = max{*ℛ*_*r*_, *ℛ*_*c*_}.

Using the parameter values given in Table 1, the sensitivity indices are listed in Tables 2 and 3 as it is given in Table 2.

Table 2 above is the summary sensitivity indices of  *ℜ*_*r*_ manipulated with parameters values from Table 1 and provides the result *ℛ*_*r*_ = 3.51  at the racism transmission rate  *α* = 1.37, which imply that racism spreads throughout the community. Moreover, sensitivity analysis given in Table 2 explains that the human population recruitment rate *Λ* and racism transmission rate *α* are highly affecting the racism reproduction number *ℜ*_*r*_.

Here, with the given parameter values in Table 3, we have computed *ℛ*_*c*_ = 6.03 at the corruption expansion rate  *β* = 1.51, which imply that corruption spreads throughout the community. Moreover, sensitivity analysis given in Table 3 explains that the human population recruitment rate *Λ* and corruption transmission rate  *β* are highly affecting the racism reproduction number *ℛ*_*c*_.

#### 4.1.1. Sensitivity Analysis Graphical Verification

In this subsection, sensitivity analysis of the racism and corruption coexistence transmission dynamics is performed to identify the most influential parameters for the spread as well as for the control of coexistence mind infection transmission in the community. The results of sensitivity analysis based on the set of parameters values given in Table 1 are analyzed in Tables 2 and 3, respectively. Graphical simulation of sensitivity indices given by Figure 2 illustrates the sensitivity index of parameters and has verified the qualitative analysis given in Tables 2 and 3, respectively. It shows that the most sensitive parameters which have direct impacts on the basic reproduction numbers are the racism transmission rate, the corruption transmission rate, and the recruitment rate and the most sensitive parameters which have an indirect impact on the basic reproduction numbers are the racism recovery rate and the corruption recovery rate. Stake holders can minimize the transmission rates and maximize recovery rates to prevent and control the coexistence expansion in the community.

### 4.2. Numerical Simulations

In this section, numerical simulation has been performed with MATAB ode45 code to analyze the effect of some parameters that causes for conducting this illegal activity. Most specifically, we investigated the stability of the endemic equilibrium point of the main coexistence model (3), parameter effects on the reproduction numbers, and the impact of being honest on racism and corruption co-acting individuals in the community. Moreover, we have used the parameters values stated in Table 1 for numerical simulation.

#### 4.2.1. Behavior of the Coexistence Model Solutions for *ℛ*_*rc*_ > 1

Figure 3 illustrates the result of numerical simulation with ode45 using parameter values that are given in Table 1. From Figure 3, we can observe that after a year the solutions of the racism and corruption coexistence dynamical system (3) will be approaching to the coexistence endemic equilibrium point of the racism-corruption coexistence model depending on the value of  *ℛ*_*rc*_ = max{*ℛ*_*r*_, *ℛ*_*c*_} = max{3.51, 6.03} = 6.03 > 1. The numerical simulation justified that the physical phenomenon that can be stated as the expansion and spreading of racism-corruption coexistence activity is consistently occurred throughout the considered community in the study.

#### 4.2.2. Impact of Racism Recovery Rate on  *ℛ*_*r*_

Figure 4 illustrates the effect of racism recovery rate *γ*_2_ on the racism reproduction number  *ℛ*_r_. The plot demonstrates that when the value of  *γ*_2_ increases, the racism reproduction number is going down, and whenever the value of *γ*_2_ > 0.059 implies that  *ℛ*_*r*_ < 1. In other words, it mean as the power of treatment rate increases the number of racial individual will decrease. Therefore, the stakeholder shall concentrate on maximizing the value of racism recovery rate *γ*_2_  by applying possible interventions strategies to prevent and control the problem of racism.

#### 4.2.3. Effect of Corruption Recovery Rate *γ*_1_ on  *ℛ*_*c*_

Figure 5 illustrates the relation between corruption recovery rate *γ*_1_ and corruption reproduction  *ℛ*_c_. The plot shows that that when the value of corruption recovery rate  *γ*_1_ increases, the corruption reproduction number decreases, and whenever the value of *γ*_1_ > 0.508 implies that  *ℛ*_*c*_ < 1. This means that as the power treatment rate increases, the number of corrupted individual decreases. Moreover, the result tells us the stakeholder shall concentrate on maximizing the values of *γ*_1_  to prevent and control the expansion of racism in the community under consideration.

#### 4.2.4. Impact of Corruption Transmission Rate *β* on  *ℛ*_c_

Figure 6 has been plotted based on the parameters values that given Table 1 which deduces the impact of corruption transmission rate *β* on the corruption reproduction number  *ℛ*_c_. The displayed simulation states that when the value of  *β*  increases, the corruption reproduction number is going up and the value of *β* < 0.17  implies that *ℛ*_*C*_ < 1. Therefore, the stakeholders are expected to minimizing the values of corruption transmission rate *β* to control corruption expansion in the community.

#### 4.2.5. Impact of Racism Transmission Rate *α* on *ℛ*_*r*_

In Figure 7, we have simulated on the relation between racism transmission rate and racism reproduction number  *ℛ*_*r*_. The plot demonstrates that whenever the value of  *α*  increases, the racism reproduction number increases, and the value of *α* < 0.322  implies that *ℛ*_*r*_ < 1. Therefore, the stakeholders are expected to minimizing the values of racism transmission rate  *α*  to control the racism expansion in the community.

#### 4.2.6. Impact of Coexistence Recovery Rate *γ*_3_ on *C*_1_

Figure 8 investigates the fact that whenever the racism-corruption recovery rate *γ*_3_  increases from 0.54 to 0.73 the number of racism-corruption co-occurrence in the community decreases. The figure deduces that when the values of *γ*_3_ increases, the number of individual conduction both racism and corruption among population is going down. This means as the power of treatment increases the racial and corrupted coexistence class in the model become decreases. Therefore, the stakeholders shall expect to maximize the values of parameter  *γ*_3_ to control the expansion of the racism-corruption coexistence in the community.

## 5. Discussion

In Section 1, we have introduced the backgrounds of the racism, corruption, and racism-corruption coexistence and reviewed some literatures related to the study. In Section 2, we have classified the total human population into seven nonmutual distinct classes and formulated the nonlinear deterministic racism and corruption coexistence dynamical system using a system of ordinary differential equations.

In Section 3, we have analyzed the qualitative behaviors of the newly developed model such as the positivity of solutions of the model, boundedness of the dynamical system, racism-free equilibrium point, and corruption-free equilibrium point. Additionally, we have analyzed the stability of endemic equilibriums, stability analysis of disease-free equilibrium point, and sensitivity analysis of reproduction numbers. We have also deduced the effect of parameters in the expansion or control of racism and corruption as well as parameter effect on the infected population.

## 6. Conclusion

Nowadays, racism and corruption coexistence is a major problem affecting nations throughout the world, but literatures on prevention and controlling its expansion through the community were rare. In this work, we have developed a first new nonlinear compartmental deterministic mathematical model on the transmission dynamics of racism and corruption coexistence expansion. The developed model has disease-free equilibrium points that are both locally asymptotically and globally asymptotically stable whenever their corresponding basic reproduction number is less than one. All the model mind infection endemic equilibrium points were both locally asymptotically and globally-asymptotically stable whenever their corresponding reproduction number is less than unity. The model did not have the phenomenon of backward bifurcation. The sensitivity analysis of the model showed us the racism transmission and corruption transmission rates are the most sensitive parameters which have a direct effect on the racism and corruption coexistence mind infection transmission in the community. Also the racism recovery rate and corruption recovery rate have high indirect impact on the basic reproduction numbers of the racism model and corruption model, respectively. Using the parameter values given in Table 1, we have obtained *ℛ*_*r*_ = 3.51 at *α* = 1.37 and *ℛ*_*c*_ = 6.03 at  *β* = 1.51, i.e.,  *ℛ*_*cr*_ = max{ *ℛ*_*r*_, *ℛ*_*c*_} = max{3.51,6.03} = 6.03. Using numerical simulation, we have verified the qualitative result that the endemic equilibrium point of the racism and corruption coexistence model is locally asymptotically stable when *ℛ*_*cr*_ = max{ *ℛ*_*r*_, *ℛ*_*c*_} = max{3.51,6.03} = 6.03 > 1. Also numerical simulation results showed that whenever the racism transmission rate increases the racism mind infection transmission increases, the corruption transmission rate increases, the corruption mind infection transmission increases, the racism recovery rate increases, the racism mind infection transmission decreases, the corruption recovery rate increases, and the corruption mind infection transmission decreases.

Moreover, based on the impact of some changes of parameters on the corresponding reproduction number  *ℛ*_*r*_ and  *ℛ*_*c*_, we shall give future directions for the stakeholders in the community. The results we have obtained have a crucial role for stakeholders, as it governs the eradication and/or persistence of racism, corruption, and racism-corruption coexistence which are illegal activities in a community. Stakeholders shall concentrate on decreasing the racism transmission rate, the corruption transmission rate, and increasing or maximizing the values of racism and corruption recovery rates that are used to minimize and possibly to eradicate the problem from the community.

Finally, we recommend the governments of nations to introduce, apply and ensure anticorruption and antidiscriminatory laws, and take the bold measures to beak the interconnection of corruption and racism. We want to remark the whole community stay unite to identify common problems and committed to research and advocacy from societies. The international institutions shall be collaborated for better understanding of these two interlinked problems and set up monitoring and investigation bodies. In the limitations of this study, the next potential researchers can incorporate them and extend this study: optimal control approach, stochastic approach, fractional order derivative approach, environmental impacts, age, and spatial structure, whenever possible validating the model by applying appropriate real data.

## Figures and Tables

**Figure 1:** Flow chart of the transmission dynamics where *λ*_*C*_ and *λ*_*R*_ are given in (1) and (2), respectively.

**Figure 2:** Parameter sensitivity analysis.

**Figure 3:** Behaviors of the coexistence model solutions.

**Figure 4:** Impact of *γ*_2_ on *ℛ*_*r*_.

**Figure 5:** Impact of *γ*_1_  on *ℛ*_c_.

**Figure 6:** Impact of *β* on  *ℛ*_c_.

**Figure 7:** Impact of *α* on *ℛ*_*r*_.

**Figure 8:** Impact of *γ*_3_ on  *C*_1_.

**Table 1:** Parameter values for numerical simulation.

Parameter	Values	Source
*μ*	0.01	[6, 12, 51]
*Λ*	50	[6, 20, 49]
*α*	Variable	Assumed
*σ*_1_	0.6	Assumed
*σ*_2_	0.7	Assumed
*η*	1.3	Assumed
*ξ*	1.2	Assumed
*θ*_3_	0.2	Assumed
*β*	Variable	Assumed
*θ*_1_	0.3	[20]
*θ*_2_	0.25	Assumed
*γ*_1_	0.007	[39, 50]
*γ*_2_	0.006	Assumed
*γ*_3_	0.008	Assumed

**Table 2:** Sensitivity indices of *ℜ*_*r*._

Sensitivity index	Sensitivity indices
SI(*Λ*)	+1
SI(*γ*_2_)	-0.85
SI(*α*)	+1

**Table 3:** Sensitivity indices of *ℜ*_*c*_.

Sensitivity index	Sensitivity indices
SI(*β*)	+1
SI(*γ*_1_)	-0.546
SI(*μ*)	-0.346
SI(*Λ*)	+1

## Data Availability

Data used to support the findings of this study are included in the article

## Appendix

### Proof of Local Stability of the Endemic Equilibrium Point of Corruption Model in the Absence of Racism (Theorem 8)

Proof To show the local stability of the endemic equilibrium point of corruption model in the absence of racism, we have used the method of Jacobian matrix and Routh-Hurwitz stability criteria. The corresponding Jacobian matrix of the dynamical system at the endemic equilibrium point *E*_*c*_^∗^ = (*S*^∗^, *C*^∗^, *R*_1_^∗^) is

(A.1) $$\begin{array}{c} J\left(\;E_{r}^{*}\right)=\left[\begin{array}{ccc} -\left(\frac{\beta }{N}C^{*}+\mu \right) & -\frac{\beta }{N}S^{*} & \theta_{1}\\ \frac{\beta }{N}C^{*} & \frac{\beta }{N}S^{*}-\left(\gamma_{1}+\mu \right) & 0\\ 0 & \gamma_{1} & -\left(\theta_{1}+\mu \right) \end{array}\right]. \end{array}$$

Then, the characteristic equation of the above Jacobian matrix is given by

(A.2) $$\begin{array}{c} \left|\begin{array}{ccc} -\left(\frac{\beta }{N}C^{*}+\mu \right)-\lambda & -\frac{\beta }{N}S^{*} & \theta_{1}\\ \frac{\beta }{N}C^{*} & \frac{\beta }{N}S^{*}-\left(\gamma_{1}+\mu \right)-\lambda & 0\\ 0 & \gamma_{1} & -\left(\theta_{1}+\mu \right)-\lambda \end{array}\right|=0,\\ \left|\begin{array}{ccc} G-\lambda & \text{H} & \theta_{1}\\ I & J-\lambda & 0\\ 0 & K & L-\lambda \end{array}\right|=0. \end{array}$$

where

(A.3) $$\begin{array}{c} \;G=-\left(\frac{\beta }{N}\left(\frac{\Lambda \lambda_{C}\left(\theta_{1}+\mu \right)}{\left(\lambda_{C}+\mu \right)\left(\theta_{1}+\mu \right)\left(\gamma_{1}+\mu \right)-\theta_{1}\gamma_{1}\lambda_{C}}\right)+\mu \right),H=-\frac{\beta }{N}\left(\frac{\Lambda \left(\theta_{1}+\mu \right)\left(\gamma_{1}+\mu \right)}{\left(\lambda_{C}+\mu \right)\left(\theta_{1}+\mu \right)\left(\gamma_{1}+\mu \right)-\theta_{1}\gamma_{1}\lambda_{C}}\right),\\ I=\frac{\beta }{N}\frac{\Lambda \lambda_{C}\left(\theta_{1}+\mu \right)}{\left(\lambda_{C}+\mu \right)\left(\theta_{1}+\mu \right)\left(\gamma_{1}+\mu \right)-\theta_{1}\gamma_{1}\lambda_{C}},J=\frac{\beta }{N}\left(\frac{\Lambda \left(\theta_{1}+\mu \right)\left(\gamma_{1}+\mu \right)}{\left(\lambda_{C}+\mu \right)\left(\theta_{1}+\mu \right)\left(\gamma_{1}+\mu \right)-\theta_{1}\gamma_{1}\lambda_{C}}\right)-\left(\gamma_{1}+\mu \right), \end{array}$$

*K* = *γ*_1_ and *L* = −(*θ*_1_ + *μ*).

(A.4) $$\begin{array}{c} \Rightarrow \lambda^{3}-\left(L+G+J\right)\lambda^{2}+\left(GL+JL+GJ-HI\right)\lambda +\left(HIL+IK\theta_{1}-LGJ\right)=0\\ \Rightarrow \left(-\left(\frac{\beta }{N}\left(\frac{\Lambda \lambda_{C}\left(\theta_{1}+\mu \right)}{\left(\lambda_{C}+\mu \right)\left(\theta_{1}+\mu \right)\left(\gamma_{1}+\mu \right)-\theta_{1}\gamma_{1}\lambda_{C}}\right)+\mu \right)-\lambda \right)\left(\frac{\beta }{N}\left(\frac{\Lambda \left(\theta_{1}+\mu \right)\left(\gamma_{1}+\mu \right)}{\left(\lambda_{C}+\mu \right)\left(\theta_{1}+\mu \right)\left(\gamma_{1}+\mu \right)-\theta_{1}\gamma_{1}\lambda_{C}}\right)-\left(\gamma_{1}+\mu \right)-\lambda \right)\left(-\left(\theta_{1}+\mu \right)-\lambda \right)+\frac{\beta }{N}\left(\frac{\Lambda \left(\theta_{1}+\mu \right)\left(\gamma_{1}+\mu \right)}{\left(\lambda_{C}+\mu \right)\left(\theta_{1}+\mu \right)\left(\gamma_{1}+\mu \right)-\theta_{1}\gamma_{1}\lambda_{C}}\right)\left(\frac{\beta }{N}\frac{\Lambda \lambda_{C}\left(\theta_{1}+\mu \right)}{\left(\lambda_{C}+\mu \right)\left(\theta_{1}+\mu \right)\left(\gamma_{1}+\mu \right)-\theta_{1}\gamma_{1}\lambda_{C}}\;\right)\left(-\left(\theta_{1}+\mu \right)-\lambda \right)+\theta_{1}\left(\left(\frac{\beta }{N}\frac{\Lambda \lambda_{C}\left(\theta_{1}+\mu \right)}{\left(\lambda_{C}+\mu \right)\left(\theta_{1}+\mu \right)\left(\gamma_{1}+\mu \right)-\theta_{1}\gamma_{1}\lambda_{C}}\right)\gamma_{1}\right)=0,\\ \Rightarrow d_{0}\lambda^{3}+d_{1}\lambda^{2}+d_{2}\lambda +d_{3}=0, \end{array}$$

where  *d*_0_ = 1 and *d*_1_ = −(*L* + *G* + *J*).

(A.5) $$\begin{array}{c} d_{1}=\left(\left(\theta_{1}+\mu \right)+\left(\gamma_{1}+\mu \right)+\left(\frac{\beta }{N}\left(\frac{\Lambda \lambda_{C}\left(\theta_{1}+\mu \right)}{\left(\lambda_{C}+\mu \right)\left(\theta_{1}+\mu \right)\left(\gamma_{1}+\mu \right)-\theta_{1}\gamma_{1}\lambda_{C}}\right)+\mu \right)-\frac{\beta }{N}\left(\frac{\Lambda \left(\theta_{1}+\mu \right)\left(\gamma_{1}+\mu \right)}{\left(\lambda_{C}+\mu \right)\left(\theta_{1}+\mu \right)\left(\gamma_{1}+\mu \right)-\theta_{1}\gamma_{1}\lambda_{C}}\right)\right),\\ \Rightarrow d_{1}=\left(\left(\theta_{1}+\mu \right)+\left(\gamma_{1}+\mu \right)+\frac{1}{N}\left(\frac{\Lambda \lambda_{C}\left(\theta_{1}+\mu \right)}{\left(\lambda_{C}+\mu \right)\left(\theta_{1}+\mu \right)-\theta_{1}\gamma_{1}\lambda_{C}}\right)\left(\left(\frac{\beta }{\left(\gamma_{1}+\mu \right)}\right)-1\right)\right),\\ \Rightarrow d_{1}=\left(\left(\theta_{1}+\mu \right)+\left(\gamma_{1}+\mu \right)+\frac{1}{N}\left(\frac{\Lambda \lambda_{C}\left(\theta_{1}+\mu \right)}{\left(\lambda_{C}+\mu \right)\left(\theta_{1}+\mu \right)-\theta_{1}\gamma_{1}\lambda_{C}}\right)\left(R_{C}-1\right)\right),\\ d_{2}=\left(GL+JL+GJ-HI\right),\\ d_{2}=\left(\left(\frac{\beta }{N}\left(\frac{\Lambda \lambda_{C}\left(\theta_{1}+\mu \right)}{\left(\lambda_{C}+\mu \right)\left(\theta_{1}+\mu \right)\left(\gamma_{1}+\mu \right)-\theta_{1}\gamma_{1}\lambda_{C}}\right)+\mu \right)\left(\theta_{1}+\mu \right)-\frac{\beta }{N}\left(\frac{\Lambda \left(\theta_{1}+\mu \right)\left(\gamma_{1}+\mu \right)\left(\theta_{1}+\mu \right)}{\left(\lambda_{C}+\mu \right)\left(\theta_{1}+\mu \right)\left(\gamma_{1}+\mu \right)-\theta_{1}\gamma_{1}\lambda_{C}}\right)-\left(\gamma_{1}+\mu \right)\left(\theta_{1}+\mu \right)+\left(\frac{\beta }{N}\left(\frac{\Lambda \lambda_{C}\left(\theta_{1}+\mu \right)}{\left(\lambda_{C}+\mu \right)\left(\theta_{1}+\mu \right)\left(\gamma_{1}+\mu \right)-\theta_{1}\gamma_{1}\lambda_{C}}\right)+\mu \right)\frac{\beta }{N}\left(\frac{\Lambda \left(\theta_{1}+\mu \right)\left(\gamma_{1}+\mu \right)}{\left(\lambda_{C}+\mu \right)\left(\theta_{1}+\mu \right)\left(\gamma_{1}+\mu \right)-\theta_{1}\gamma_{1}\lambda_{C}}\right)-\left(\gamma_{1}+\mu \right)\right),\\ \Rightarrow d_{2}=\frac{\beta }{N}\left(\frac{\Lambda \lambda_{C}\left(\theta_{1}+\mu \right)}{\left(\lambda_{C}+\mu \right)\left(\theta_{1}+\mu \right)\left(\gamma_{1}+\mu \right)-\theta_{1}\gamma_{1}\lambda_{C}}\right)\left(\left(\theta_{1}+\mu \right)\left(\frac{\beta }{\left(\gamma_{1}+\mu \right)}\right)-1\right),\\ \Rightarrow d_{2}=\frac{\beta }{N}\left(\frac{\Lambda \lambda_{C}\left(\theta_{1}+\mu \right)}{\left(\lambda_{C}+\mu \right)\left(\theta_{1}+\mu \right)\left(\gamma_{1}+\mu \right)-\theta_{1}\gamma_{1}\lambda_{C}}\right)\left(\left(\theta_{1}+\mu \right)\right)\left(R_{C}-1\right). \end{array}$$

Finally, by following the same algebraic manipulation,  *d*_3_ = (*HIL* + *IKθ*_1_ − *LGJ*).

(A.6) $$\begin{array}{c} \;d_{3}=\left(HIL+IK\theta_{1}-LGJ\right),\\ \Rightarrow d_{3}=\left(\frac{\beta }{N}\left(\frac{\Lambda \left(\theta_{1}+\mu \right)\left(\gamma_{1}+\mu \right)}{\left(\lambda_{C}+\mu \right)\left(\theta_{1}+\mu \right)\left(\gamma_{1}+\mu \right)-\theta_{1}\gamma_{1}\lambda_{C}}\right)\;\left(\frac{\beta }{N}\frac{\Lambda \lambda_{C}\left(\theta_{1}+\mu \right)}{\left(\lambda_{C}+\mu \right)\left(\theta_{1}+\mu \right)\left(\gamma_{1}+\mu \right)-\theta_{1}\gamma_{1}\lambda_{C}}\;\right)\left(\theta_{1}+\mu \right)+\left(\frac{\beta }{N}\frac{\Lambda \lambda_{C}\left(\theta_{1}+\mu \right)}{\left(\lambda_{C}+\mu \right)\left(\theta_{1}+\mu \right)\left(\gamma_{1}+\mu \right)-\theta_{1}\gamma_{1}\lambda_{C}}\right)\gamma_{1}\theta_{1}+\left(\theta_{1}+\mu \right)\left(\frac{\beta }{N}\left(\frac{\Lambda \left(\theta_{1}+\mu \right)\left(\gamma_{1}+\mu \right)}{\left(\lambda_{C}+\mu \right)\left(\theta_{1}+\mu \right)\left(\gamma_{1}+\mu \right)-\theta_{1}\gamma_{1}\lambda_{C}}\right)-\left(\gamma_{1}+\mu \right)\right)\left(\frac{\beta }{N}\left(\frac{\Lambda \lambda_{C}\left(\theta_{1}+\mu \right)}{\left(\lambda_{C}+\mu \right)\left(\theta_{1}+\mu \right)\left(\gamma_{1}+\mu \right)-\theta_{1}\gamma_{1}\lambda_{C}}\right)+\mu \right)\right),\\ \Rightarrow d_{3}=\left(\left(\frac{\beta }{N}\frac{\Lambda \lambda_{C}\left(\theta_{1}+\mu \right)}{\left(\lambda_{C}+\mu \right)\left(\theta_{1}+\mu \right)\left(\gamma_{1}+\mu \right)-\theta_{1}\gamma_{1}\lambda_{C}}\;\right)\left(\theta_{1}+\mu \right)\right)\left(\frac{\beta }{N}\left(\frac{\Lambda \left(\theta_{1}+\mu \right)\left(\gamma_{1}+\mu \right)}{\left(\lambda_{C}+\mu \right)\left(\theta_{1}+\mu \right)\left(\gamma_{1}+\mu \right)-\theta_{1}\gamma_{1}\lambda_{C}}\right)+\left(\frac{\beta }{\left(\gamma_{1}+\mu \right)}\right)-1\right),\\ \Rightarrow d_{3}=\left(\left(\frac{\beta }{N}\frac{\Lambda \lambda_{C}\left(\theta_{1}+\mu \right)}{\left(\lambda_{C}+\mu \right)\left(\theta_{1}+\mu \right)\left(\gamma_{1}+\mu \right)-\theta_{1}\gamma_{1}\lambda_{C}}\;\right)\left(\theta_{1}+\mu \right)\right)+\left(\frac{\beta }{N}\left(\frac{\Lambda \left(\theta_{1}+\mu \right)\left(\gamma_{1}+\mu \right)}{\left(\lambda_{C}+\mu \right)\left(\theta_{1}+\mu \right)\left(\gamma_{1}+\mu \right)-\theta_{1}\gamma_{1}\lambda_{C}}\right)\left(R_{C}-1\right)\right). \end{array}$$

From the above algebraic manipulation, all the coefficients of the characteristic's polynomial are positives whenever  *ℛ*_*c*_ > 1. Therefore, by applying Routh-Hurwitz, we have the following array for the polynomial *d*_0_*λ*^3^ + *d*_1_*λ*^2^ + *d*_2_*λ* + *d*_3_ = 0.

(A.7) $$\begin{array}{c} \begin{array}{c} \lambda^{3}\\ \lambda^{2}\\ \lambda^{1}\\ \lambda^{0} \end{array}\left|\begin{array}{cc} d_{0} & d_{2}\\ d_{1} & d_{3}\\ e_{1} & 0\\ {\text{f}}_{1} & 0 \end{array}\right., \end{array}$$

where

(A.8) $$\begin{array}{c} e_{1}=\frac{-1}{d_{1}}\left|\begin{array}{cc} d_{0} & d_{2}\\ d_{1} & d_{3} \end{array}\right|=\frac{-1}{d_{1}}\left(d_{0}d_{3}-d_{1}d_{2}\right)=e_{1}=\frac{-1}{d_{1}}\left(d_{0}d_{3}-d_{1}d_{2}\right),\\ e_{1}=\frac{-1}{d_{1}}\left(d_{3}-d_{1}d_{2}\right)=\left(\left(\frac{\beta }{N}\frac{\Lambda \lambda_{C}\left(\theta_{1}+\mu \right)}{\left(\lambda_{C}+\mu \right)\left(\theta_{1}+\mu \right)\left(\gamma_{1}+\mu \right)-\theta_{1}\gamma_{1}\lambda_{C}}\;\right)\left(\theta_{1}+\mu \right)\right)+\left(\frac{\beta }{N}\left(\frac{\Lambda \left(\theta_{1}+\mu \right)\left(\gamma_{1}+\mu \right)}{\left(\lambda_{C}+\mu \right)\left(\theta_{1}+\mu \right)\left(\gamma_{1}+\mu \right)-\theta_{1}\gamma_{1}\lambda_{C}}\right)\left(R_{C}-1\right)\right)+\left(\left(\theta_{1}+\mu \right)+\left(\gamma_{1}+\mu \right)+\frac{1}{N}\left(\frac{\Lambda \lambda_{C}\left(\theta_{1}+\mu \right)}{\left(\lambda_{C}+\mu \right)\left(\theta_{1}+\mu \right)-\theta_{1}\gamma_{1}\lambda_{C}}\right)\left(\left(\frac{\beta }{\left(\gamma_{1}+\mu \right)}\right)-1\right)\right)\left(\left(\frac{\beta }{N}\left(\frac{\Lambda \lambda_{C}\left(\theta_{1}+\mu \right)}{\left(\lambda_{C}+\mu \right)\left(\theta_{1}+\mu \right)\left(\gamma_{1}+\mu \right)-\theta_{1}\gamma_{1}\lambda_{C}}\right)+\mu \right)\left(\theta_{1}+\mu \right)+\left(\frac{\beta }{N}\left(\frac{\Lambda \lambda_{C}\left(\theta_{1}+\mu \right)}{\left(\lambda_{C}+\mu \right)\left(\theta_{1}+\mu \right)\left(\gamma_{1}+\mu \right)-\theta_{1}\gamma_{1}\lambda_{C}}\right)+\mu \right)\frac{\beta }{N}\left(\frac{\Lambda \left(\theta_{1}+\mu \right)\left(\gamma_{1}+\mu \right)}{\left(\lambda_{C}+\mu \right)\left(\theta_{1}+\mu \right)\left(\gamma_{1}+\mu \right)-\theta_{1}\gamma_{1}\lambda_{C}}\right)\right)>0\text{ for }R_{C}>1,\\ \Rightarrow e_{1}>0. \end{array}$$

Following the same procedure,

(A.9) $$\begin{array}{c} f_{1}=\frac{-1}{e_{1}}\left|\begin{array}{cc} d_{1} & d_{3}\\ e_{1} & e_{1} \end{array}\right|=\frac{-1}{e_{1}}\left(e_{1}d_{1}-d_{3}e_{1}\right),\\ \Rightarrow f_{1}=\left(\left(\left(\frac{\beta }{N}\frac{\Lambda \lambda_{C}\left(\theta_{1}+\mu \right)}{\left(\lambda_{C}+\mu \right)\left(\theta_{1}+\mu \right)\left(\gamma_{1}+\mu \right)-\theta_{1}\gamma_{1}\lambda_{C}}\;\right)\left(\theta_{1}+\mu \right)\right)\left(\left(\frac{\beta }{N}\frac{\Lambda \lambda_{C}\left(\theta_{1}+\mu \right)}{\left(\lambda_{C}+\mu \right)\left(\theta_{1}+\mu \right)\left(\gamma_{1}+\mu \right)-\theta_{1}\gamma_{1}\lambda_{C}}\;\right)\left(\theta_{1}+\mu \right)\right)\left(\frac{\beta }{N}\left(\frac{\Lambda \left(\theta_{1}+\mu \right)\left(\gamma_{1}+\mu \right)}{\left(\lambda_{C}+\mu \right)\left(\theta_{1}+\mu \right)\left(\gamma_{1}+\mu \right)-\theta_{1}\gamma_{1}\lambda_{C}}\right)+\left(R_{C}-1\right)\right)\right)>0\text{ for }R_{C}>1,\\ \Rightarrow f_{1}>0. \end{array}$$

We have observed that the first column of the Routh-Hurwitz array has no sign change; thus, the endemic equilibrium point of the dynamical system is locally asymptotically stable if *ℛ*_*C*_ > 1.

## Abbreviations

### Symbols

*μ*: Natural death rate
*Λ*: The recruitment rate
*θ*_2_: The rate at which racism removed individuals who lose their honesty
*θ*_3_: The rate at which racism and corruption coexistence removed individuals loss their honesty
*θ*_1_: The rate at which corruption removed individuals who lose their honesty
*σ*_1_: The rate at which racial and corrupted individuals recovered from racism and become corrupted only
*γ*_1_: The rate at which corrupted individuals stop doing corruption
*ξ*: Modification parameter
*σ*_2_: The rate at which racial and corrupted individuals recovered from corruption and become racial only.
*η*: Modification parameter
*γ*_2_: The rate at which racial individuals stop participating in the act of racism
*γ*_3_: The rate at which racial and corrupt coexistence individuals stop the act of racism and corruption.

### Variables

*S*: Susceptible individuals
*C*: Individuals who are corrupt
*R*: Individuals who are racial
*C*_1_: Individuals who participate in both racism and corruption
*R*_1_: Individuals who stop participating in corruption
*R*_2_: Individuals who stop the act of racism
*R*_3_: Individuals who are removed from both racism and corruption and become honest
